The article "Bee venom-loaded EGFR-targeting peptide-coupled chitosan nanoparticles for effective therapy of hepatocellular carcinoma by inhibiting EGFR-mediated MEK/ERK pathway" was retracted in 2023. Reasons: concerns about the data; concerns about the images.

# Bee venom-loaded EGFR-targeting peptide-coupled chitosan nanoparticles for effective therapy of hepatocellular carcinoma by inhibiting EGFR-mediated MEK/ERK pathway

**DOI:** 10.1371/journal.pone.0272776

**Published:** 2022-08-10

**Authors:** Shaymaa Abdulmalek, Nouf Mostafa, Marwa Gomaa, Mohamed El‑Kersh, Ayman I. Elkady, Mahmoud Balbaa

**Affiliations:** 1 Department of Biochemistry, Faculty of Science, Alexandria University, Alexandria, Egypt; 2 Plant Protection Research Institute, Agriculture Research Center, Giza, Egypt; 3 Zoology Department, Faculty of Science, Alexandria University, Alexandria, Egypt; Centre de Recherche en Biologie cellulaire de Montpellier, FRANCE

## Abstract

Hepatocellular carcinoma (HCC) is one of the world’s most risky diseases due to the lack of clear and cost-effective therapeutic targets. Currently, the toxicity of conventional chemotherapeutic medications and the development of multidrug resistance is driving research into targeted therapies. The nano-biomedical field’s potential for developing an effective therapeutic nano-sized drug delivery system is viewed as a significant pharmaceutical trend for the encapsulation and release of numerous anticancer therapies. In this regard, current research is centered on the creation of biodegradable chitosan nanoparticles (CSNPs) for the selective and sustained release of bee venom into liver cancer cells. Furthermore, surface modification with polyethylene glycol (PEG) and GE11 peptide-conjugated bee venom-CSNPs allows for the targeting of EGFR-overexpressed liver cancer cells. A series of *in vitro* and *in vivo* cellular analyses were used to investigate the antitumor effects and mechanisms of targeted bee venom-CSNPs. Targeted bee venom-CSNPs, in particular, were found to have higher cytotoxicity against HepG2 cells than SMMC-7721 cells, as well as stronger cellular uptake and a substantial reduction in cell migration, leading to improved cancer suppression. It also promotes cancer cell death in EGFR overexpressed HepG2 cells by boosting reactive oxygen species, activating mitochondria-dependent pathways, inhibiting EGFR-stimulated MEK/ERK pathway, and elevating p38-MAPK in comparison to native bee venom. In hepatocellular carcinoma (HCC)-induced mice, it has anti-cancer properties against tumor tissue. It also improved liver function and architecture without causing any noticeable toxic side effects, as well as inhibiting tumor growth by activating the apoptotic pathway. The design of this cancer-targeted nanoparticle establishes GE11-bee venom-CSNPs as a potential chemotherapeutic treatment for EGFR over-expressed malignancies. Finally, our work elucidates the molecular mechanism underlying the anticancer selectivity of targeted bee venom-CSNPs and outlines therapeutic strategies to target liver cancer.

The article "Bee venom-loaded EGFR-targeting peptide-coupled chitosan nanoparticles for effective therapy of hepatocellular carcinoma by inhibiting EGFR-mediated MEK/ERK pathway" was retracted in 2023. Reasons: concerns about the data; concerns about the images.

## Introduction

Cancer is still one of the top leading causes of mortality worldwide, accounting for millions of deaths each year. Mainly, hepatocellular carcinoma (HCC) is one of the most prevalent liver tumors, with a high rate of recurrence and metastasis [1]. In addition, the efficacy of the standard cytotoxic drugs is poor, necessitating the development of new therapeutic targets. Since conventional anti-cancer drugs utilized in chemotherapy cannot always exhibit predominant tumor specificity related to normal cells. Chemotherapy-based new drug system design, particularly targeted drug delivery systems, has become one of the most widely used methods for cancer treatment. Remarkably, the boosted permeability and retention effect of nanotechnology-based drug delivery as well as the surface modification of nanoparticles for specific targeting of tumor cells, has emerged to offer more effective delivery of drugs to tumors by binding to a specific receptor.

Receptor crosstalk has gotten a lot of attention in recent years as a key component in comprehending the increasingly complicated signaling networks that operate within normal and cancer cells. The epidermal growth factor receptor (EGFR) system appears to operate as a signaling core where numerous extracellular survival and growth signals converge [2]. EGFR belongs to the receptor tyrosine kinase family (RTKs). When EGFR binds to its ligands in the epidermal growth factor (EGF) family, it dimerizes and leads to conformational activation of the tyrosine kinase domain (TKD), which then phosphorylates key tyrosine residues in the c-terminal tail of EGFR [3]. EGFR has emerged as a critical therapeutic target in the treatment of cancer [4, 5]. Overexpression of EGFR is common in HCC, suggesting that it may have a role in the development and therapy of the disease [6]. The interaction of anticancer drugs specifically with the cancer cells is considered to be particularly significant for the selection of anti-cancer drugs to achieve the most efficient cancer therapy. Consequently, anti-EGFR-targeted therapy may provide a therapeutic power or provide a breakthrough in the treatment of HCC. Here, the synthetic GE11 peptide (12-amino-acid), with the sequence YHWYGYTPQNVI, is an effective peptide for targeting EGFR, making it one of the best options for the development of EGFR-targeted drug delivery systems [7].

Interestingly, in traditional medicine, bee venom derived from honeybees is often used to treat disorders such as arthritis, skin diseases, and tumors [8, 9]. It is made up of a complex mix of biologically active peptides, such as melittin (a major component of bee venom), apamin, and phospholipase A2, all of which have different pharmaceutical properties. Many studies have shown that natural extracts, such as venoms/toxins obtained from bees, snakes, and scorpions have anticancer properties [10]. Recently, research has discovered that bee venom possesses anti-cancer properties, such as inducing apoptosis and inhibiting proliferation in cancer cells from the prostate, liver, ovarian, breast, lung, and bladder [11–13]. The synergistic effect and selective cytotoxicity of melittin appear to be responsible for bee venom’s efficacy [14].

The article "Bee venom-loaded EGFR-targeting peptide-coupled chitosan nanoparticles for effective therapy of hepatocellular carcinoma by inhibiting EGFR-mediated MEK/ERK pathway" was retracted in 2023. Reasons: concerns about the data; concerns about the images.

Therapeutically, chitosan has been employed as a polymer-based nano-drug platform(s) in numerous biomedical applications for the delivery of a variety of drug types for the treatment of cancers [15, 16]. Chitosan has a slow circulatory pattern and a low immunological clearance rate [17]. Furthermore, chitosan can enter the epithelial membranes’ tight junction efficiently, resulting in better permeability through this junction. Surface modifications of chitosan, besides its physicochemical properties, play a central role in the cytotoxic profile and targeting of tumors with rapid division and aggressive growth [18]. In addition to this, polyethylene glycol (PEG) is a hydrophilic-based synthetic polymer that has been employed in a variety of pharmacotherapeutic applications. FDA has approved it as a biodegradable polymer that is non-immunogenic and non-antigenic for use in biological applications [19]. As a result, it’s frequently utilized as an encapsulating or coating agent in nanoparticle-based drug delivery systems.

In this study, we used chitosan nanoparticles (CSNPs) conjugated with PEG and GE11 to encapsulate and transport bee venom for the treatment of HCC. The targeted bee venom-loaded GE11 conjugated CSNPs may improve bee venom’s cytotoxicity against cancer cells. This work investigated the *in vitro* cellular uptake process and anticancer activity of targeted bee venom-CSNPs, as well as the underlying molecular mechanisms. As well, assessed the role of targeted bee venom-CSNPs on EGFR-mediated tyrosine kinase cascades; MEK/ERK, and p38-MAPK to support the rationale for applying natural compounds-based nanomaterials in clinical trials for cancer therapy. Besides *in vivo* investigation of the antitumor efficiency and systemic toxicity of targeted bee venom-CSNPs on HCC-induced mice.

## Materials and methods

### Materials

Human liver cancer HepG2 and SMMC-7721 cells were purchased from American Type Culture Collection (ATCC, Manassas, Virginia, USA). Dimethyl sulfoxide (DMSO) and Annexin V/fluorescein isothiocyanate (FITC) apoptosis detection kit was purchased from (Cell signaling technology, Beverly, MA, USA). Chitosan (purity ≥ 98%), EDC, dialysis bags (MWCO: 8000–14,000), Polyethylene glycol (PEG), acetic acid 100%, Diethyl nitrosamine (DEN), and Carbon tetrachloride (CCL_4_) were obtained from (Sigma-Aldrich, St. Louis, MO, USA). Dulbecco’s Modified Eagle Medium (DMEM), ROS kit, 0.25% tryp-sin-EDTA, Fetal bovine serum, penicillin-streptomycin, and GE11 polypeptide were purchased from Gibco, Thermo Fisher Scientific, Inc. (Waltham, MA, USA). Additionally, 3-(4, 5-dimethylthiazol-2-yl)-2, 5-diphenyltetrazolium bromide (MTT), bicinchoninic acid (BCA) protein assay kit, paraformaldehyde, and coumarin-6, were purchased from (Sigma-Aldrich, St. Louis, MO, USA). SensiFAST SYBR Green No-ROX Kit (BIO-98005) and SensiFAST cDNA Synthesis kit (BIO-65054) (Meridian Bioscience, Cincinnati, OH, USA), QIAzol Lysis Reagent (#79306) (QIAGEN, Hilden, Germany). RIPA lysis buffer, Bcl-2 (4223) antibody, Bax (2774) antibody, p-EGFR (3777) antibody, p-p38-MAPK (9211) anti-body, p-p38-MAPK (9215) antibody, ERK (9102) antibody, p-ERK (4377) antibody, MEK (9122), p-MEK (9154) antibody, β-actin (4970) antibody, and anti-rabbit IgG were purchased from the Cell signaling technology (Beverly, MA, USA). Erlotinib (≥ 98%) and U0126 (≥ 98% pure) were purchased from Merck and Co., Inc. (Kenilworth, NJ, United States).

The article "Bee venom-loaded EGFR-targeting peptide-coupled chitosan nanoparticles for effective therapy of hepatocellular carcinoma by inhibiting EGFR-mediated MEK/ERK pathway" was retracted in 2023. Reasons: concerns about the data; concerns about the images.

### Collection of bee venom

This work was carried out in the Department of Apiculture, Plant Protection Research Institute, Agriculture Research Center, Sakha, Kafr El-Sheikh, during the 2019 summer season. Venom was collected from the honeybee (Apis mellifera L.) workers of the pure Carniolan race as well as its hybrid with 1-, 2-, 3-, and 4-week intervals in two experiments of collections by different methods (fiber and latex) [20, 21]. Bee workers were stimulated to sting through latex or fiber sheets put on a glass plate using electrical impulses, and the dry venom was collected using a pointed scraper. Bees that came into contact with the wires were stung on the glass sheet and suffered a slight electrical shock. The alarm odor from the venom mobilized and angered the other bees, and they began to sting as well. The venom gathered by the bees dries on the glass. For transit to the laboratory, the frames with fresh dried bee venom are carefully placed into a specific container. The processing of bee venom begins as soon as the frames are returned to the laboratory. After that, the bee venom is sealed in dark glass jars and stored in a cool, dry location [22].

### The analysis results of bee venom sample using HPLC single-point calibration method

HPLC analysis was performed using an Agilent 1260 series. The separation was performed using stainless steel column (25cm*4.8mm) packed with octadecylsilyl silica gel for chromatography (5μm) (nucleosil C18 is suitable). The mobile phase consisted of (A) 0.1% trifluoroacetic acid and (B) acetonitrile at a flow rate of 1 ml/min. The wavelength detector was observed at 345 nm. For each of the sample solutions, the injection volume was 20 μl for 60 min. The column temperature was maintained at 35°C. The samples and standards were prepared by dissolving 1 mg in 1 ml Milli-Q water then sonicated for 10 min then diluted with (95A/5B) mobile phase.

The article "Bee venom-loaded EGFR-targeting peptide-coupled chitosan nanoparticles for effective therapy of hepatocellular carcinoma by inhibiting EGFR-mediated MEK/ERK pathway" was retracted in 2023. Reasons: concerns about the data; concerns about the images.

### Preparation of targeted bee venom-chitosan nanoparticles

Chitosan nanoparticles (CSNPs) have been fabricated using the ionotropic gelation technique. Then the aqueous solution of Polyethylene glycol (PEG) (5%) was prepared using a simple stirring speed of around 500 rpm for 30 min at room temperature. After dissolving PEG in acidic chitosan solution, it was left to be mixed for 30 min with a stirring speed of 250 rpm. Then bee venom solution was added to the CSNPs-PEG mixture. The drug copolymers were left for 1 h within a mild stirring speed. Finally, tripolyphosphate (TPP) was added to allow sufficient cross-linking between bee venom and the other polymers. The solutions were kept mixing under mild stirring conditions for 30 min. The formulated CSNPs were directly separated by using ultracentrifugation at 10,000 rpm for 30 min. Then the dialysis against Milli-Q water was used to eliminate the excess reactants. After that, the prepared bee venom-CSNPs were further combined with 40 μl, 500 mM EDC solution to activate the COOH group on the surfaces of bee venom-loaded PEGylated CSNPs and 80 μl GE11 peptide solution for an overnight reaction at 4°C to obtain targeted bee venom-CSNPs. Then the dialysis against Milli-Q water was used to remove the excess reactants. All the preparation processes were repeated to get coumarin 6-loaded nanoparticles, by adding 100 μl coumarin-6 solution to the mixture of CSNPs, and then the surface of prepared nanoparticles was modified with GE11 peptide.

### Characterization of morphology, size, and surface charge of prepared nanoparticles

Transmission electron microscopy (TEM) and Dynamic Light Scattering (DLS) techniques were used to examine the morphology, surface properties, and size of the synthesized targeted bee venom-CSNPs. The bee venom-CSNPs solution was placed onto the copper net and allowed to dry for 12 h at room temperature. TEM images were captured by using the TEM instrument (JEOL JEM-1400Flash, Tokyo, Japan). DLS was used to measure the size distribution and zeta potential of the nanoparticles (DLS, Malvern Instruments, Malvern, United Kingdom).

The article "Bee venom-loaded EGFR-targeting peptide-coupled chitosan nanoparticles for effective therapy of hepatocellular carcinoma by inhibiting EGFR-mediated MEK/ERK pathway" was retracted in 2023. Reasons: concerns about the data; concerns about the images.

### Determination of entrapment efficiency

The amount of bee venom encapsulated in the nanoparticles was determined by subtracting the total amounts of venom added in the nanoparticle preparation solution from the amount of non-entrapped venom remaining in the clear supernatant, which was measured at 595 nm using the Bradford method after centrifugation at 11,000 rpm and 4°C for 90 min [23]. The following equation was used to compute the venom entrapment efficiency (EE) of nanoparticles: % EE = [(A-B)/A] 100, where A represents total venom and B represents free venom.

### Nanoparticles *in vitro* stability test

Targeted bee venom-CSNPs samples were suspended in buffer solution, pH 7.4 at 4°C for 30 days to investigate long-term *in vitro* stability (storage stability). The purpose of the test is to stress the stability of nanoparticles to obtain data for a pharmaceutical product formulation study. At predetermined time intervals, the sizes and dispersion of nanoparticles were measured. Moreover, after 30 days of incubation, the morphology of targeted bee venom-CSNPs in buffer solution was confirmed by TEM.

### *In vitro* release study

At 37°C and 200 rpm, several tubes containing 3 mg of freeze-dried bee venom-CSNPs and 3 ml of phosphate buffer (PBS), 0.2 mol/l, pH 7.4 were shaken. At the relevant time intervals (1, 2, 4, 6, 17, 24, 30, and 48 h), a single tube was withdrawn and centrifuged for 30 min at 11,000 rpm and 4°C. The amount of bee venom released in the supernatant was determined using the Bradford protein assay spectrophotometric technique at 595 nm [23]. The total released protein concentration at each time point was estimated using a standard curve.

### Cell culture

HepG2 and SMMC-7721 cells were obtained from the American Type Culture Collection (USA). Dulbecco’s Modification of Eagle’s Medium (DMEM) supplemented with 10% fetal bovine serum, 4 mM l-glutamine, 50 U penicillin/ml, and 50 g streptomycin/ml was used as the culture media in a humidified incubator at 37°C and set to 5% CO_2_. 10% dimethyl sulfoxide (DMSO) in fetal bovine serum was used as the freezing medium. Phosphate-buffered saline (PBS), pH was adjusted to 7.4 and stored for a maximum of 6 months at 4°C.

### Cell cytotoxicity assay

HepG2 and SMMC-7721 cells (1×10^5^) were cultured in DMEM supplemented with 10% FBS and kept at 37°C in a humidified 5% CO_2_ incubator. The 3-(4,5-dimethylthiazol-2-yl)-2,5-diphenyltetrazolium bromide (MTT) colorimetric test was used to measure cell proliferation. The cells were seeded at a density of 2×10^3^ cells/well in 96-well culture plates. After a 24 h incubation period, different quantities of each treatment (CSNPs, Bee venom, non-targeted CSNPs, and targeted bee venom-CSNPs) were introduced to each well at 6.25, 12.5, 25, 50, and 100 μg/ml. After 24 h, each well was filled with 50 μl of MTT solution (2 mg/ml) added to each well, then incubated for 4 h. The culture media was withdrawn and an equal volume of DMSO was added to each well to dissolve formazan crystals. MTT is converted into a purple-colored formazan product with an absorbance maximum near 570 nm by viable cells with an active metabolism. The absorbance of each well was determined at a wavelength of 570 nm using ELISA reader (LERX-800 Biotek–USA). The viability percent was calculated as follows: Viability % = Mean OD Treated X 100/Mean OD Control. Where OD is optical density. The IC_50_ is the concentration of the used drug required to induce 50% inhibition of cell growth and the value was calculated by fitting the survival curve using graph pad prism software [24].

The article "Bee venom-loaded EGFR-targeting peptide-coupled chitosan nanoparticles for effective therapy of hepatocellular carcinoma by inhibiting EGFR-mediated MEK/ERK pathway" was retracted in 2023. Reasons: concerns about the data; concerns about the images.

### Cellular uptake and *in vitro* imaging studies

The cellular uptake and distribution modifications of targeted bee venom-CSNPs into HepG2 and SMMC-7721 cells were studied using fluorescent microscopy. Overnight, about 1×10^5^ HepG2 cells were grown in a 6-well plate in serum-containing DMEM media. The cells were then loaded with coumarin 6-loaded nanoparticles and incubated for 0.5, 1, 1.5, 2, 3, and 6 h after being washed once with PBS. Related cells were collected and rinsed twice with PBS. After fixed time intervals, related cells were collected and washed twice with EDTA-free PBS solution. Then, for cell lysis, 50 μl of 0.5% Triton X-100 in NaOH (0.2 N) was added to each well. Finally, the fluorescence intensity of the collected cells was measured using a microplate reader with 430 nm excitation wavelength and 485 nm emission wavelength. Moreover, the photo images of cells were taken by fluorescent microscopy (ZOETM Fluorescent Cell Imager, Bio-Rad, Hercules, CA, USA).

### Anti-EGFR antibody blocking assay and peptide competition assay

HepG2 cells were seeded at a density of 1×10^5^ cells/well in 96 well plates for a free EGFR-peptide competition experiment. Excess EGFR-peptide concentrations were added to the wells and incubated for 1 h. The cells were then incubated for 2 h with coumarin-6-loaded targeted bee venom-CSNPs. In addition to this, HepG2 cells were placed into 96 well plates at a density of 1×10^5^ cells/well for 24 h, then anti-EGFR antibody was added and incubated for 1 h. The cells were then incubated for 0.5, 1, and 2 h with coumarin-6-loaded targeted bee venom-CSNPs. Cells were then washed and lysed in a 0.2 M NaOH solution containing Triton X-100 (0.5%). The fluorescence intensity of coumarin-6-loaded targeted bee venom CSNPs inside the wells was measured using a fluorescent microplate reader with excitation and emission wavelengths of 430 and 485 nm, respectively.

The article "Bee venom-loaded EGFR-targeting peptide-coupled chitosan nanoparticles for effective therapy of hepatocellular carcinoma by inhibiting EGFR-mediated MEK/ERK pathway" was retracted in 2023. Reasons: concerns about the data; concerns about the images.

### Cell migration assay

HepG2 and SMMC-7721 cells were seeded at a density of 2×10^5^ cells/well in 6-well culture plates and grown to 100% confluence. 200 μl pipette tip was used in a sterile environment to press firmly against the top of the tissue culture plate and make a vertical wound down through the confluent cell monolayer, and each well was washed with PBS to remove non-adherent cells. The media and cell debris were aspirated carefully. Then, against the well wall, enough culture media was added to cover the bottom of the well and prevent additional cells from detaching. The first photograph was then taken. The tissue culture plate was incubated at 37°C and 5% CO_2_. The cells were treated with targeted bee venom-CSNPs and then incubated for 30 h. The perimeter of the central cell-free zone was confirmed under a microscope. Images were captured at 0 and 30 h using a microscope at X100 magnification and the area of the wound was quantified using ImageJ 1.47v software (http://imagej.nih.gov/ij). The migration of cells was evaluated from the width of the wounded area [25].

### Colony formation assay

Assays for colony development were carried out as previously described. HepG2 and SMMC-7721 cells were seeded at a concentration of 500 cells per well in 6-well plates and left to grow overnight. The cells were then incubated for 2 h with targeted bee venom-CSNPs. After removing the drug-containing media, the cells were washed in PBS and cultured for another 10 days in a complete medium to form colonies. After that, the cells were rinsed twice with PBS and fixed with 2% paraformaldehyde. Then 1 ml of (1%, 25 mM) crystal violet was added to each well of 6-well plates containing fixed colonies and incubated at room temperature for 30 min. The dye was removed, and the wells were rinsed twice with PBS and then three times with dH_2_O. Cell colonies with more than 25 cells were manually counted in five magnification fields at random, and the results were expressed as a percentage of the control. At least three separate tests were carried out [26, 27].

### DNA fragmentation study

The amount of DNA fragmentation caused by the biosynthesized nanoparticles was measured using agarose gel electrophoresis. HepG2 cells were treated with bee venom, targeted bee venom-CSNPs, and non-targeted CSNPs. Centrifugation at 3000 rpm for 15 min at 4°C was used to separate the treated and untreated cells. The cell pellet was lysed for 10 min at 4°C in a lysis solution containing 10 mmol/l Tris-HCl pH 7.4, 10 mmol/l EDTA, and 0.5% Triton X-100. The lysates were centrifuged at 20,000 rpm for 20 min before being treated for 1 h at 37°C with 200 mg/ml RNase A and 200 mg/ml proteinase K. Following chloroform extraction, the samples were extracted with phenol/chloroform/isoamyl alcohol (25:24:1, v/v/v). In two volumes of ice-cold ethanol, DNA was precipitated in the presence of 0.3 mol/l sodium acetate. After drying, DNA was dissolved in Tris/EDTA buffer and separated on a 1.5% agarose gel electrophoresis, with gel documentation (ChemiDoc™ Imaging System, Bio-Rad, Hercules, CA, USA) used to check for DNA damage [28].

The article "Bee venom-loaded EGFR-targeting peptide-coupled chitosan nanoparticles for effective therapy of hepatocellular carcinoma by inhibiting EGFR-mediated MEK/ERK pathway" was retracted in 2023. Reasons: concerns about the data; concerns about the images.

### Apoptosis analysis by flow cytometry

According to the manufacturer’s recommendations, the apoptotic cell distribution was assessed using the Annexin V/Dead Cell Kit. Briefly, after HepG2 treatments with bee venom, targeted bee venom-CSNPs, and non-targeted CSNPs, all cells were collected and diluted to a concentration of 5×10^5^ cells/ml in PBS containing 1% bovine serum albumin (BSA) as a dilution buffer. In a microtube, 100 μl of Annexin V/Dead Cell reagent and 100 μl of a single cell suspension were combined and incubated at room temperature for 20 min in the dark. After that, the cells were examined using the BD FACSLyric (San Jose, CA, USA).

### Measurement of intracellular ROS

HepG2 cells were extracted, washed twice in PBS, centrifuged, and suspended in PBS. Subsequently, the cells were then stained with the ROS detection kit at 37°C for 30 min following the manufacturer’s instructions. After that, the cells were then incubated for various periods at 37°C with targeted bee venom-CSNPs, non-targeted CSNPs, or bee venom (100 μl/well). The level of intracellular ROS was measured using a microplate reader to assess cell fluorescence intensity (excitation and emission wavelength set as 485 and 530 nm).

### RNA extraction, cDNA synthesis, and real-time PCR

HepG2 cells were seeded into 25 cm^2^ flasks (TPP-Swiss) at a density of 1×10^5^ cells/ml. Cancer cells were treated with the IC_50_ for 24 h and an untreated flask was considered. The cells that were affected were collected, and the rest of the cells were trypsinized and centrifuged at 4°C. Pelted cells were rinsed in PBS and transferred to Eppendorf tubes as before. Total RNA was extracted according to the manufacturer’s instructions using QIAzol Lysis Reagent. Spectrophotometry was used to check the quality of RNA samples. RNAs of high quality were kept at -80°C until they were needed. The SensiFAST cDNA synthesis kit was used to create cDNA products from RNA according to the manufacturer’s instructions. The reaction mixture was run in a thermal cycler (Bio-Rad, Hercules, CA, USA). SensiFAST SYBR Green Kit was used to accomplish quantitative real-time PCR gene quantification. The real-time PCR primers for Bcl-2 were as follows: F: 5ʹ-ATGTGTGTGGAGACCGTCAA-3ʹ and R: 5ʹ- GCCG-TACAGTTCCACAAAGGG -3ʹ. The Bax real-time PCR primers were F: 5ʹ- ATGTTTTCTGACGGCAACTTC -3ʹ and R: 5ʹ- AGTCCAATGTCCAGCCCAT -3ʹ. The caspase-9 real-time PCR primers were F: 5ʹ- CATTTCATGGTG-GAGGTGAAG-3ʹ and R: 5ʹ- GGGAACTG-CAGGTGGCTG -3ʹ. The caspase-3 real-time PCR primers were F: 5ʹ-TGTTTGTGTGCTTCTGAGCC-3ʹ and R: 5ʹ-CACGCCATGTCATCATCAAC -3ʹ. GAPDH was used as an endogenous control gene for the quantitative reverse transcription–PCR assay. The sequence of the primers for reference gene GAPDH was F: 5ʹ-GGCACAGTCAAGGCTGAGAATG-3ʹ and 5′ R: 5ʹ- ATGGTGGTGAAGACGCCAGTA -3ʹ [29].

The article "Bee venom-loaded EGFR-targeting peptide-coupled chitosan nanoparticles for effective therapy of hepatocellular carcinoma by inhibiting EGFR-mediated MEK/ERK pathway" was retracted in 2023. Reasons: concerns about the data; concerns about the images.

### Protein extraction and western blot analysis

For western blotting, about 1×10^5^ HepG2 cells were plated in 6-well culture plates. The media was withdrawn, and the cells were washed twice with ice-cold PBS before being lysed with RIPA cell lysis buffer with a protease inhibitor cocktail. Scraping the lysates from the plates was followed by centrifugation at 12,000 g for 5 min at 4°C. Protein concentrations were assessed using the BCA protein assay method and an equal volume of total proteins was examined on 12% SDS-PAGE after denaturation at 95°C for 10 min in the presence of 80 mM Dithiothreitol (DTT). Proteins were transferred to PVDF membranes by Mini-Trans Blot (Bio-Rad, Hercules, CA, USA) after electrophoresis, and membranes were blocked with 5% skim milk before incubation overnight with primary antibodies p-ERK1/2, ERK1/2, p-p38MAPK, p38MAPK, p-EGFR, p-MEK, MEK, Bcl-2, Bax and β-actin. The membranes were then treated with HRP-conjugated secondary antibodies before being detected using the TMB-western blot kit. ImageJ 1.47v software (http://imagej.nih.gov/ij) was used to examine the bands. The intensity values for the proteins of interest were normalized using β-actin protein level as a reference [30].

### *In vivo* study

The animal experiment design protocol was approved by the ethics committee of animal research in Pharmaceutical and Fermentation Industries Development Center, (SRTA-City), Egypt, Institutional Animal Care and Use Committees (IACUC)/IACUC#30-1Y-1021. Seventy male Swiss albino mice, fifteen-day-old were obtained from Alexandria University Medical Research Institute’s laboratory animal house, Egypt, following the institute’s animal care policy. The mice were kept in polycarbonate cages with stainless-steel wire tops, with five mice per cage. The mice were kept in a typical environment with a temperature of 25°C, relative humidity of 70%, and a 12-hour light-dark cycle. Throughout the studies, the animals were fed ordinary pellets and free access to tap water.

The article "Bee venom-loaded EGFR-targeting peptide-coupled chitosan nanoparticles for effective therapy of hepatocellular carcinoma by inhibiting EGFR-mediated MEK/ERK pathway" was retracted in 2023. Reasons: concerns about the data; concerns about the images.

### Induction of hepatocellular carcinoma

The mice were randomly allocated. Healthy control (n = 8): mice were injected intraperitoneally with normal saline at the time of treatment of other groups. HCC-induced (n = 8): mice were intraperitoneally injected with 70 mg/kg body weight of DEN weekly followed by intramuscular injection of carbon tetrachloride (CCl_4_) (0.5 ml/kg body weight, with an equal amount of olive oil) for 8 weeks. Three mice were chosen at random from the control and induced groups and blood was taken through heart puncture at week four after the induction process. The level of blood alpha-fetoprotein (AFP), a tumor marker for HCC, was then tested using an ELISA kit. Following confirmation of the AFP level mice were divided randomly into five treatment groups as follow; Bee venom 1 mg/kg (n = 8): HCC-mice injected intraperitoneally with freshly prepared 1 mg/kg bee venom; Bee venom 2 mg/kg (n = 8): HCC-mice injected intraperitoneally with freshly prepared 2 mg/kg bee venom; Targeted bee venom-CSNPs 0.5 mg/kg (n = 8): HCC-mice injected intraperitoneally with freshly prepared 0.5 mg/kg targeted bee venom-CSNPs; Targeted bee venom-CSNPs 1 mg/kg (n = 8): HCC-mice injected intraperitoneally with freshly prepared 1 mg/kg targeted bee venom-CSNPs; Non-targeted CSNPs 2 mg/kg (n = 8): HCC-mice injected intraperitoneally with freshly prepared 2 mg/kg non-targeted CSNPs. All current treatment options were administered to mice daily for four weeks. At the end of the experimental period and after twenty-four hours of last treatment, mice were fasted overnight and sacrificed after being anesthetized with sodium pentobarbital (100 mg/kg). Blood was collected from caudal vena cava, kept at room temperature for 15 min, then centrifuged at 3000 rpm for 10 min and serum was stored at -20°C until used. Livers were removed immediately, and small portions were fixed in 10% formalin for histopathological examination. The liver was washed with a cold saline solution and kept at -80°C.

### Serum biochemical assays

The assays of liver function enzymes such as Alanine transaminase (ALT), Aspartate transaminase (AST), alkaline phosphatase (ALP), albumin, and total protein were performed in the serum of mice using commercial kits (Spectrum Diagnostics, Egypt), also serum alpha-fetoprotein was determined by using mouse-specific ELISA kit Mybiosource (MBS033826) and according to manufacturer instructions.

### Real-Time Polymerase Chain Reaction (RT-PCR)

Total RNA was extracted from frozen liver using QIAzol Lysis Reagent, as directed by the manufacturer. Primer sequence (Sigma-Aldrich): Bcl-2, F:5ʹ-ATGTGTGTGGAGACCGTCAA-3ʹ and R: 5ʹ-GCCGTACAGTTCCACAAAGGG-3ʹ; Bax, F:5ʹ-ATGGAGCTGCAGAGGATGATT-3ʹ and R:5ʹ-TGAAGTTGCCATCAGCAAACA-3ʹ; Caspase-9, F:5ʹ-CATTTCATGGTGGAGGTGAAG-3ʹ and R:5ʹ-GGGAACTGCAGGTGGCTG-3ʹ; Caspase-3, F:5ʹ-AATTCAAGGGACGGGTCATG-3ʹ and R:5ʹ-GCTTGTGCGCGTACAGTTTC-3ʹ; MMP-9, F: 5′-TGTACCGCTATGGTTACACTCG-3′ R:5′-GGCAGGGACAGTTGCTTCT-3′; MMP-2, F:5′-TTGACGGTAAGGACGGACTC-3′ R:5′- CATACTTCACACGGAC-CACTTG-3′; GAPDH, F:5ʹ-GGCACAGTCAAGGCTGAGAATG-3ʹ and R:5ʹ- ATGGTGGTGAAGACGCCAGTA -3ʹ.

The article "Bee venom-loaded EGFR-targeting peptide-coupled chitosan nanoparticles for effective therapy of hepatocellular carcinoma by inhibiting EGFR-mediated MEK/ERK pathway" was retracted in 2023. Reasons: concerns about the data; concerns about the images.

### Histopathological study

Dehydration in escalating grades of alcohol was used to dehydrate the fixed liver tissues in 10% formalin, followed by impregnation. After that, the sections were embedded in paraffin and left to sit at room temperature. Serial pieces of 5 μm thick were cut using a rotatory microtome. Following that, sections were stained with Haematoxylin and Eosin (H&E) and histological alterations were identified [31].

### Statistical analyses

Statistical analyses were performed with GraphPad Prism v8 (GraphPad Software Inc.), Office Excel 365 (Microsoft), and SPSS Predictive Analytics Software (IBM, Version 26). All data were derived from multiple experiments conducted at least in triplicate. For multiple comparison data, one-way ANOVA followed by Tukey’s post-hoc test was used to make individual comparisons and p < 0.01 were statistically significant.

## Results

### HPLC analysis of bee venom

HPLC was used to identify the primary components of collected bee venom. The standard melittin, phospholipase 2, apamin retention times, and linear lines were determined to compare them to the component of the tested bee venom gathered from bees. **Table 1 and Fig 1** illustrate the retention time (RT), concentration, and area under the curve (AUC) of the standard bee venom and prepared sample mixture.

**Fig 1:** Chromatogram of bee venom. (**A**) Standard mixture; and (**B**) Sample mixture.

**Table 1:** HPLC single-point calibration method for the analysis results of the bee venom sample.

	Bee Venom sample mixture	Bee Venom standard mixture
**RT**	47.29	47.12
**Area**	20,104.33	15,522.33
**Concentration**	**75**	**58.07**

### Preparation and characterization of targeted bee venom-CSNPs

**Fig 2** shows transmission electron microscope micrographs of CSNPs, non-targeted CSNPs, and targeted bee venom-CSNPs prepared at optimum concentrations (1 mg/ml CS and 1 mg/ml TPP for CSNPs, and 1 mg/ml CS and 1 mg/ml TPP with 300 μg/ml of bee venom) with particle size of 34, 56, and 80 nm, respectively. The nanoparticles had smooth surfaces and an almost spherical form (**Fig 2A**). In addition, the average particle size and distribution of the nanoparticles were measured by DLS. The average size of CSNPs was 43.8 nm with a PDI (0.24±0.01), while the average size of non-targeted CSNPs was 78.8 nm with a PDI (0.12±0.001), and the targeted bee venom-CSNPs was 122 nm with a PDI (0.11±0.002) (**Fig 2B**). The entrapment efficiency of prepared bee venom nanoparticles was 88.65%. Moreover, the data illustrated the zeta potentials of non-targeted CSNPs and targeted bee venom-CSNPs, which were prepared at optimum concentrations (1 mg/ml CS with 300 μg/ml of venom). The values of zeta potentials were 6.61 and 2.3 mV of non-targeted CSNPs and targeted bee venom-CSNPs, respectively (**Fig 2C**). Besides, *in vitro* release of the bee venom-CSNPs was assessed using the nanoparticles that were prepared at the optimum concentrations with 89% of encapsulation efficiency for bee venom-CSNPs. The releasing behavior of prepared nanoparticles, according to the data, roughly 85% of the loaded venom was released within 48 h of incubation in phosphate buffer solution (PBS), pH 7.4. The venom release profile showed a 45% burst release in the first seven hours, followed by a gradual release during the next 30 h (**Fig 2D**).

The article "Bee venom-loaded EGFR-targeting peptide-coupled chitosan nanoparticles for effective therapy of hepatocellular carcinoma by inhibiting EGFR-mediated MEK/ERK pathway" was retracted in 2023. Reasons: concerns about the data; concerns about the images.

**Fig 2:** Characterization of prepared nanoparticles. (**A**) Transmission electron microscope image; (**B**) particle size; (**C**) Zeta potential; (**D**) Release profile of bee venom from CSNPs relative to time.

#### Nanoparticles *in vitro* stability

Targeted bee venom-CSNPs were initially resuspended in physiologic PBS buffer (pH 7.4) and stored at 4°C to assess the nanoparticle suspension’s storage stability as a potential parenteral formulation. At predefined time intervals, the diameters of nanoparticles and their size distribution were measured for 30 days. At all experimental time settings, shows good stability for prepared targeted bee venom-CSNPs, with no significant increases in size or PDI (p<0.01, **Table 2**). In addition, after 30 days, the synthesized nanoparticles had a round shape and good sizes, as compared to the morphology of the nanoparticles before the incubation period (**Fig 3A and 3B**). These characteristics suggest that our nanoparticulate platform could be a good candidate for obtaining prolonged stability.

**Fig 3:** TEM micrographs of (**A**) fresh prepared targeted bee venom-CSNPs and (**B**) targeted bee venom-CSNPs after 30 days incubation in a buffer.

**Table 2:** Size and PDI changes of targeted bee venom-CSNPs stored in buffer solution at 4°C.

Time (days)	Particle size (nm)	PDI
**0**	122±0.50	0.11±0.002
**1**	122±0.45	0.13±0.001
**5**	123±0.33	0.13±0.002
**10**	120±0.65	0.24±0.001
**13**	115±0.56	0.21±0.002
**15**	110±0.43	0.22±0.002
**20**	117±0.34	0.32±0.002
**22**	125±0.58	0.11±0.001
**26**	121±0.53	0.14±0.001
**28**	122±0.45	0.17±0.001
**30**	121±0.55	0.16±0.001

Values are expressed as mean ± SE, (n = 3). Statistical analyses were performed using one-way ANOVA.

The article "Bee venom-loaded EGFR-targeting peptide-coupled chitosan nanoparticles for effective therapy of hepatocellular carcinoma by inhibiting EGFR-mediated MEK/ERK pathway" was retracted in 2023. Reasons: concerns about the data; concerns about the images.

### Enhanced selectivity of anticancer activity of targeted bee venom-CSNPs

The MTT assay was used to evaluate the inhibitory effect of bee venom, CSNPs, non-targeted CSNPs, and targeted bee venom-CSNPs on cell growth in human liver cancer HepG2 and SMMC-7721 cells. In a dose-dependent manner (100, 50, 25, 12.5, and 5 g/ml), bee venom alone significantly suppressed the development of HepG2 and SMMC-7721 cells compared to control cells. The combination of bee venom and CSNPs enhanced the effect of bee venom on cancer cell proliferation, and the targeted bee venom-CSNPs showed a dramatic inhibitory effect on cell growth of HepG2 due to overexpression of the EGFR receptor than SMMC-7721 cells, demonstrating its strong proliferation-inhibition effects. The inhibitory concentration (IC_50_) of targeted bee venom-CSNPs was 22.25 μg/ml and 59.77 μg/ml for HepG2 and SMMC-7721 cells, respectively. While IC_50_ of non-targeted CSNPs was 127.54 μg/ml and 181.51 μg/ml for HepG2 and SMMC-7721 cells, respectively. And IC_50_ of native bee venom was 77.72 μg/ml and 85.29 μg/ml for HepG2 and SMMC-7721 cells, respectively. Also, data showed that CSNPs recorded the lowest inhibitory effect on the viability of tested cancer cell lines compared with bee venom and venom-loaded nanoparticles that, IC_50_ value was 349.36 μg/ml and 852.89 μg/ml for HepG2 and SMMC-7721 cells, respectively, **Fig 4**. Taking all of the data into account, using a specific peptide targeted EGFR as a carrier for bee venom could be a very effective technique to improve its efficacy and selectivity against cancer cells.

**Fig 4:** Cell viability of HepG2 and SMMC-7721. Relationship between targeted bee venom-CSNPs, non-targeted CSNPs, native bee venom, and CSNPs concentrations and viability percentage on HepG2 and SMMC-7721 cells.

### Cellular uptake of targeted bee venom-CSNPs

The intracellular fluorescence of coumarin-6-loaded bee venom-CSNPs was detected using a microplate reader to assess the cellular uptake of targeted bee venom-CSNPs in both HepG2 and SMMC-7721 cells. Obtained results demonstrated that the uptake of targeted bee venom-CSNPs nanoparticles in HepG2 cells was high, reaching 100% uptake after 6 h incubation, while the results of SMMC-7721 cells, which has a middle EGFR expression and showed lower uptake than HepG2 cells, reaching 72% after 6 h incubation (**Fig 5A**). On the other hand, the uptake of non-targeted CSNPs in HepG2 and SMMC-7721 cells were 39.6 and 30.7%, respectively after 6 h incubation (**Fig 5B**).

The article "Bee venom-loaded EGFR-targeting peptide-coupled chitosan nanoparticles for effective therapy of hepatocellular carcinoma by inhibiting EGFR-mediated MEK/ERK pathway" was retracted in 2023. Reasons: concerns about the data; concerns about the images.

**Fig 5:** Cellular uptake of bee venom-loaded CSNPs. (**A**) Cellular uptake of coumarin-6-loaded targeted bee venom nanoparticles in HepG2 and SMMC-7721 cells; (**B**) coumarin-6-loaded non-targeted nanoparticles in HepG2 and SMMC-7721 cells, n = 3.

### EGFR expression and selective cellular uptake of coumarin-6 loaded targeted bee venom-CSNPs

Firstly, we compared the expression of EGFR in HepG2 and SMMC-7721 cells. According to the results of the western blot analysis (**Fig 6A**), EGFR was expressed most significantly in HepG2 cells and least strongly in SMMC-7721 cells. As a result, HepG2 cells with high EGFR expression were chosen to investigate the particular targeting impact of targeting bee venom-CSNPs mediated by GE11 peptides further. We evaluated the internalization of couramin-6 loaded targeted bee venom-CSNPs in EGFR high expressed HepG2 cells and EGFR medium expressed SMMC-7721 cells (**Fig 6B**) to examine the selectivity of targeted bee venom-CSNPs. We used an EGFR-specific peptide competing for assay in HepG2 and SMMC-7721 cells to further investigate the role of EGFR-specific peptide in the absorption of coumarin-6-loaded targeted bee venom-CSNPs. The cells were pretreated with an excess of the peptide before being incubated with coumarin-6-loaded targeted bee venom-CSNPs for a variety of times. Free GE11 peptide could considerably block cellular uptake of targeted bee venom-CSNPs, as shown in **Fig 6B**, and 4 mg/ml GE11 peptide administration resulted in roughly 40% lower uptake of coumarin-6-loaded targeted bee venom-CSNPs. Anti-EGFR antibody was also employed to block EGFR in HepG2 cells, resulting in a nearly 30% reduction in coumarin-6-loaded GE11-bee venom-CSNPs absorption (**Fig 6C**). These findings suggested that cancer cells’ selective cellular uptake of targeted bee venom-CSNPs may be related in part to EGFR-dependent endocytosis.

**Fig 6:** EGFR expression and selective cellular uptake of targeted bee venom-CSNPs. (**A**) EGFR expression; (**B**) selective cellular uptake of coumarin-6 loaded targeted bee venom-CSNPs; (**C**) and anti-EGFR antibody blocking in HepG2 and SMMC-7721 cells.

### Inhibition of cell migration and colony formation by targeted bee venom-CSNPs

A wound-healing assay was used to assess migration. HepG2 and SMMC-7721 cells were treated with non-targeted CSNPs and targeted bee venom-CSNPs supplemented with 1% FBS in the wound-healing assay. When compared to untreated cells, the diameter of the wound had a lesser propensity for closure after 15 and 30 h. After 30 h, untreated HepG2 and SMMC-7721 cells filled the wounded area, whereas, in the targeted bee venom-CSNPs-treated cells, a distinct gap remained, and the width of the gaps was greater in HepG2-treated cells than SMMC-7721-treated cells, **Fig 7A**. In addition to this, the colony formation experiment was performed on HepG2 and SMMC-7721 cells to further assess the effects of targeted bee venom-loaded CSNPs on cancer cell growth. Targeted bee venom-loaded CSNPs inhibited colony formation in HepG2 cells more effectively than SMMC-7721 cells treated with targeted bee venom-CSNPs, which had a moderate effect on colony formation when compared to HepG2-treated cells, **Fig 7B**.

The article "Bee venom-loaded EGFR-targeting peptide-coupled chitosan nanoparticles for effective therapy of hepatocellular carcinoma by inhibiting EGFR-mediated MEK/ERK pathway" was retracted in 2023. Reasons: concerns about the data; concerns about the images.

**Fig 7:** Migration ability of HepG2 and SMMC-7721 cells. (**A**) wound-healing assays; (**B**) colony formation in HepG2 and SMMC-7721 cells treated with targeted bee venom-CSNPs.

### Induction of apoptosis and overproduction of ROS in targeted bee venom-CSNPs-treated HepG2 cells

In our work, HepG2 cells with high EGFR expression were chosen to further investigate the specific targeting impact of targeted bee venom-CSNPs compared to native bee venom. Annexin-V FITC/PI apoptosis assays were used to confirm the apoptotic effect of targeted bee venom-CSNPs on HepG2 cells. Targeted bee venom-CSNPs caused apoptosis in HepG2 cells, according to the findings. **Fig 8A** shows that when HepG2 cells were treated with targeted bee venom-CSNPs, the number of apoptotic cells increased when compared to native bee venom and non-targeted CSNPs, indicating that cell death induced by targeted bee venom-CSNPs was primarily caused by apoptosis. For targeted bee venom-CSNPs, the early apoptotic cell proportions in the lower right quadrant (FITC+/PI−) were 49.82%. The late apoptotic or necrotic cell proportions in the upper right quadrant (FITC+/PI+) were 39.7 and 2.47%, respectively. These results suggest that targeted bee venom-CSNPs partially inhibited the proliferation of HepG2 cells via the induction of apoptosis. Too, we measured the ROS level after targeted bee venom-CSNPs treatment since bee venom is an anticancer drug that induces cancer cell apoptosis in a ROS-dependent manner. **Fig 8B** shows that targeted bee venom-CSNPs increased ROS formation in HepG2 cells after 5 min of treatment, followed by a gradual decrease after 60 min. It’s worth noting that targeted bee venom-CSNPs produced more ROS than native bee venom, implying this combination of targeted bee venom-CSNPs synergistically increased intracellular ROS levels in HepG2 cells, resulting in greater anticancer activity. We additionally looked into the induction of apoptosis in HepG2 cells via the occurrence of DNA fragmentation. DNA collected from untreated HepG2 cells showed no fragmentation, whereas DNA extracted from cells treated with targeted bee venom-CSNPs showed DNA laddering, which was caused by endonuclease action at sites between nucleosomes (**Fig 8C**).

The article "Bee venom-loaded EGFR-targeting peptide-coupled chitosan nanoparticles for effective therapy of hepatocellular carcinoma by inhibiting EGFR-mediated MEK/ERK pathway" was retracted in 2023. Reasons: concerns about the data; concerns about the images.

**Fig 8:** Studying the effects of targeted bee venom-CSNPs, non-targeted CSNPs, or native bee venom on induction of cell apoptosis. (**A**) Flow cytometry analysis; (**B**) ROS; and (**C**) DNA fragmentation in HepG2 treated cells.

### Cancer cell apoptosis induced by targeted bee venom-CSNPs

**Table 3** summarizes the results of real-time PCR analysis of gene expression levels for pre-and anti-apoptotic Bax, caspase 9, caspase 3, and Bcl-2 genes in HepG2 cells, where it was noticed that Bax, caspase 9, and caspase 3 genes showed a significant up-regulation in gene expression after treatment with native bee venom, but the extreme up-regulation of Bax, caspase 9, and caspase 3 expressions showed in targeted bee venom-loaded CSNPs more than other treatments. On the other hand, Bcl-2 exhibited a marked downregulation of gene expression with maximum inhibition in targeted bee venom-loaded CSNPs.

**Table 3:** Effect of non-targeted CSNPs and targeted bee venom-loaded CSNPs on Bcl-2, Bax, caspase 9, and caspase 3 genes expression in HepG2 cells.

Groups	Relative expression of genes			
	Bax	Bcl-2	Caspase-9	Caspase-3
**Non-treated HepG2 cells**	3.5±0.01 ^d^	144.56±3.55 ^a^	0.047±0.001 ^c^	0.04±0.002 ^d^
**Bee Venom-treated cells**	455.54±4.66 ^b^	33.60±1.54 ^c^	3.52±0.21 ^a^	79.15±3.54 ^b^
**Non-targeted CSNPs**	147.05±3.87 ^c^	88.28±2.70 ^b^	1.08±0.16 ^b^	3.34±0.27 ^c^
**Targeted bee venom-CSNPs**	887.75±4.65 ^a^	14.65±1.15 ^d^	4.74±0.23 ^a^	1902.01±10.54 ^a^

Values are expressed as mean ± SE, (n = 3), means for the same parameter with different letters in each bar are significantly different (p < 0.01), where the highest data value takes the letter (a).

### Activation of intracellular apoptotic pathways and inhibition of EGFR-mediated tyrosine kinase pathways by targeted bee venom-CSNPs

The mitochondrial respiratory chain is the primary source of intracellular ROS synthesis, implying that aberrant ROS production could be caused by mitochondrial dysfunction. Bcl-2 proteins and homologs regulate mitochondrial outer membrane permeabilization, which can be classified as pro-apoptotic or anti-apoptotic. Bcl-2 is a key anti-apoptotic protein in the Bcl-2 family, while Bax is a key pro-apoptotic protein, and both are involved in mitochondria-dependent apoptosis. As shown in **Fig 9A**, we discovered that treating HepG2 cells with targeted bee venom-CSNPs reduced Bcl-2 expression while increasing Bax expression, indicating that mitochondrial dysfunction was also implicated in the targeted bee venom-CSNPs inhibited HepG2 cells. Overexpression and phosphorylation of EGFR, which are prevalent mechanisms in epithelial malignancies, are linked to poor prognosis, metastasis, and chemotherapy resistance, making it a suitable target for cancer therapy. We then looked at EGFR expression and phosphorylation, finding that targeted bee venom-CSNPs suppressed EGFR phosphorylation more than bee venom alone or non-targeted CSNPs (**Fig 9B**). Briefly, the effect of targeted bee venom-CSNPs treatment on the expression levels of tyrosine kinases was investigated to confirm if this signaling pathway participates in the regulation of apoptosis. The protection of cells against apoptosis is tightly linked to the activation of the EGFR-downstream MEK/ERK signaling pathway. We also discovered that targeted bee venom-CSNPs inhibited the phosphorylation of MEK and ERK using western blot analysis, demonstrating that targeted bee venom-CSNPs could inhibit the EGFR-mediated MEK/ERK pathway, which is a key signal transduction pathway of cell proliferation with upregulation of p38-MAPK phosphorylation. These findings suggested that targeted bee venom-CSNPs promoted cell death in HepG2 cells by blocking EGFR-mediated MEK/ERK and activating p38-MAPK (**Fig 9C**).

The article "Bee venom-loaded EGFR-targeting peptide-coupled chitosan nanoparticles for effective therapy of hepatocellular carcinoma by inhibiting EGFR-mediated MEK/ERK pathway" was retracted in 2023. Reasons: concerns about the data; concerns about the images.

**Fig 9:** Activation of mitochondria-dependent apoptosis pathway and regulation of EGFR-mediated p38-MAPK/MEK/ERK pathway by targeted bee venom-CSNPs. (**A**) Western blot analysis for the expression of Bcl-2 and Bax in HepG2 cells; (**B**) Western blot analysis for the expression of p-EGFR; (**C**) Western blot analysis for the expression of p38MAPK, p-p38MAPK, MEK, p-MEK, ERK, and p-ERK; (**D**) HepG2 cells were treated with targeted bee venom-CSNPs and/or U0126 for 24 h, and the protein levels of p-ERK1/2 and total ERK1/2 were detected; (**E**) HepG2 cells were treated with targeted bee venom-CSNPs and/or Erlotinib for 24 h, and the protein levels of p-EGFR and total EGFR were detected. β-Actin was used as a loading control. Data are expressed as mean ± SEM (n = 3), means for the same parameter with different letters in each bar are significantly different (p < 0.01), where the highest data value takes the letter (a).

Current findings show that the targeted bee venom-CSNPs exhibited a considerable suppression of phosphorylation of ERK1/2, as assessed (**Fig 9C**). The reduction in pERK1/2 protein levels was validated with the use of ERK selective inhibitor, U0126. We measured total and phosphorylated ERK expression after 24 h of treatment with targeted bee venom-CSNPs or/and U1026. As shown in **Fig 9D**, there are no significant differences in total ERK protein levels between targeted bee venom-CSNPs alone and targeted bee venom-CSNPs plus 10 μM U0126 therapy. Conversely, when targeted bee venom-CSNPs and/or U0126 were given alone or together, ERK1/2 phosphorylation was significantly reduced, with a maximum inhibition of ERK1/2 phosphorylation in HepG2 cells treated with combined therapy of targeted bee venom-CSNPs and U0126. These results indicate the possibility of ERK involvement in the pathology of liver cancer, suggesting the role of targeted bee venom-CSNPs as an ERK inhibitor as well.

The article "Bee venom-loaded EGFR-targeting peptide-coupled chitosan nanoparticles for effective therapy of hepatocellular carcinoma by inhibiting EGFR-mediated MEK/ERK pathway" was retracted in 2023. Reasons: concerns about the data; concerns about the images.

Also, our results showed that targeted bee venom-CSNPs suppress the phosphorylation of EGFR and its downstream pathway molecules, which control cell proliferation, as shown in **Fig 9B and 9C**. When targeted bee venom-CSNPs were given alone or combined with Erlotinib, an inhibitor of EGFR tyrosine kinase, the inhibitory effect on EGFR phosphorylation was increased significantly (**Fig 9E**). From the above results, our findings suggested that targeted bee venom-CSNPs may have a potential utility in the treatment of liver cancer since it inhibits both EGFR and its downstream targets MEK/ERK.

### Level of serum liver enzymes in HCC mice

Induction of HCC for 2 months considerably increased the activities of ALT and AST compared to those in normal mice, implying that DEN administration may cause harm to the liver’s functional activity. Nonetheless, when compared to untreated mice, all the therapies utilized in our investigation demonstrated a considerable reduction in serum ALT and AST levels. Supplementation of targeted bee venom-CSNPs resulted in a greater reduction in ALT and AST levels compared to untreated mice (p < 0.01). Furthermore, when compared to the untreated group, the activity of ALP was dramatically reduced following therapy. Furthermore, when HCC-induced mice were compared to control healthy mice, total protein and albumin levels were found to be significantly lower. After treatments, especially with targeted bee venom-CSNPs, the values were close to control healthy mice (**Table 4**). Moreover, following HCC induction, the amount of AFP, a tumor marker, was significantly raised in mice. When compared to untreated mice, the level of AFP in all groups was significantly lower after therapy. Interestingly, treatment of induction groups with targeted bee venom-CSNPs at a dose (1 mg/kg) resulted in a more significant decrease in AFP levels than other treatments (**Table 4**).

**Table 4:** Biomarkers f serum liver function in all treated groups of HCC-induced mice.

Groups	ALT (U/L)	AST (U/L)	ALP (U/L)	Albumin (mg/dl)	Alpha-Fetoprotein (ng/ml)
**Control healthy**	35.60±1.07 ^c^	33.60±1.00 ^e^	90.51±1.71 ^d^	4.08±0.25 ^a^	09.40±0.31 ^f^
**HCC-induced**	194.29±2.25 ^a^	199.88±3.01 ^a^	198.02±2.46 ^a^	2.00±0.07 ^c^	400.60±8.43 ^a^
**Bee venom (1 mg/kg)**	39.40±1.02 ^c^	90.22±1.06 ^c^	130.66±1.83 ^c^	2.82±0.28 ^b^	100.80±3.59 ^c^
**Bee venom (2 mg/kg)**	42.08±1.10 ^c^	55.28±1.08 ^d^	90.50±1.07 ^d^	3.26±0.13 ^b^	45.20±1.37 ^d^
**Targeted bee venom-CSNPs (0.5 mg/kg)**	30.62±1.29 ^d^	47.21±0.88 ^d^	88.08±1.65 ^d^	3.34±0.10 ^b^	26.80±1.37 ^e^
**Targeted bee venom-CSNPs (1 mg/kg)**	36.08±1.07 ^c^	33.28±1.19 ^e^	72.88±1.19 ^e^	4.00±0.18 ^a^	15.80±0.77 ^f^
**Non-targeted CSNPs (2 mg/kg)**	90.06±2.08 ^b^	101.84±2.52 ^b^	164.66±2.02 ^b^	2.44±0.05 ^c^	308.60±6.62 ^b^

Results are represented as mean ± SEM (n = 8). Statistical analyses were performed using one-way ANOVA; means for the same parameter with different letters (a-f) in each column are significantly different (p < 0.01), where the highest data value takes the letter (a).

The article "Bee venom-loaded EGFR-targeting peptide-coupled chitosan nanoparticles for effective therapy of hepatocellular carcinoma by inhibiting EGFR-mediated MEK/ERK pathway" was retracted in 2023. Reasons: concerns about the data; concerns about the images.

### Induction of apoptosis by targeted bee venom-CSNPs

The results of gene expression levels for pro-apoptotic Bax, caspase 9, caspase 3, and anti-apoptotic Bcl-2 genes in HCC-induced mice revealed that Bax, caspase 9, and caspase 3 were significantly downregulated, while Bcl-2 was significantly upregulated, compared to normal groups. However, as compared to untreated groups and following our treatments, the expression levels of Bax, caspase 9, and caspase 3 were dramatically elevated especially in groups treated with targeted bee venom-CSNPs compared with native bee venom. Whereas Bcl-2 gene expression was significantly reduced in groups treated with targeted bee venom-CSNPs compared with native bee venom. In addition, when HCC-induced groups were treated, the level of liver MMP-9 and MMP-2 gene expression was significantly higher than in the control groups. MMP-9 and MMP-2 levels were found to be significantly lower in induced animals given different treatments with more efficient results in targeted bee venom-CSNPs-treated groups than in native bee venom-treated mice (**Table 5**).

**Table 5:** Effect of targeted bee venom-CSNPs and native bee venom on Bcl-2, Bax, caspase 9, caspase 3, MMP-9, and MMP-2 genes expression.

Groups	Relative expression of genes					
	Bcl-2	Bax	Caspase-9	Caspase-3	MMP-2	MMP-9
**Control healthy**	1.00±00	1.00±00	1.00±00	1.00±00	1.00±00	1.00±00
**HCC-induced**	50.18±4.45 ^a^	0.75±0.02 ^e^	0.24±0.02 ^f^	0.13±0.01 ^f^	30.10±2.43 ^a^	11.10±2.43 ^a^
**Bee venom (1 mg/kg)**	18.37±1.06 ^c^	2.69±1.02 ^c^	1.69±0.04 ^d^	1.24±0.20 ^d^	20.89±0.23 ^b^	9.89±0.23 ^b^
**Bee venom (2 mg/kg)**	10.00±1.23 ^d^	3.64±1.11 ^c^	2.42±0.08 ^c^	2.55±0.93 ^c^	15.65±3.26 ^c^	8.65±3.26 ^c^
**Targeted bee venom-CSNPs (0.5 mg/kg)**	3.04±0.38 ^e^	8.02±1.23 ^b^	10.23±0.08 ^b^	5.44±1.01 ^b^	10.97±2.47 ^d^	3.97±2.47 ^d^
**Targeted bee venom-CSNPs (1 mg/kg)**	0.89±0.07 ^f^	31.09±3.43 ^a^	17.89±1.23 ^a^	12.75±1.13 ^a^	1.81±0.021 ^e^	0.71±0.021 ^e^
**Non-targeted CSNPs (2 mg/kg)**	32.18±2.21 ^b^	1.46±0.65 ^d^	1.02±1.23 ^e^	0.58±0.23 ^e^	23.59±0.03 ^b^	9.59±0.03 ^b^

Results are represented as mean ± SEM (n = 8). Statistical analyses were performed using one-way ANOVA; means for the same parameter with different letters (a-e) in each column are significantly different (p < 0.01), where the highest data value takes the letter (a).

The article "Bee venom-loaded EGFR-targeting peptide-coupled chitosan nanoparticles for effective therapy of hepatocellular carcinoma by inhibiting EGFR-mediated MEK/ERK pathway" was retracted in 2023. Reasons: concerns about the data; concerns about the images.

### Histopathology

To observe the effect of targeted bee venom-CSNPs and native bee venom on histopathological alterations in the liver tissue of HCC-induced rats, we detected the modifications in each structure of liver tissue with H&E staining. As shown in **Fig 10A**, the liver of the control healthy displays normal hepatocytic cords with normal hepatic cells and a clear central vein. On the other hand, as shown in **Fig 10B**, a liver section of HCC-induced showing complete hepatocellular carcinoma with complete loss of the normal architecture with trabecular growth, most of the hepatic tissue is necrotic and occupied by mononuclear cells infiltration and pyknotic nucleus with the degenerated area, which is occupied by centrilobular congestion and congested dilated portal tracts along with hemorrhage, also some hepatocytes with rounded nuclei and vacuolated cytoplasm are seen. The treatment with 2 doses of native bee venom showed loss of the normal architecture with a focal area of hepatic necrosis occupied by the pyknotic nucleus and a large, degenerated area, which is occupied by centrilobular congestion and congested dilated portal tracts along with hemorrhage and some hepatocytes with rounded nuclei and vacuolated cytoplasm are seen (**Fig 10C and 10D**). Conversely, treatment of HCC-induced mice with targeted bee venom-CSNPs showing central vein with some hemorrhage and almost normal hepatocytes with some hepatocytes suffer from vacuolar and hydropic degeneration (**Fig 10E and 10F**). but non-targeted-CSNPs not showed any improvement in liver sections and the liver lost its normal architecture with a focal area of hepatic necrosis occupied by the pyknotic nucleus and a larger degenerated area occupied by centrilobular congestion and congested dilated portal tracts along with hemorrhage (**Fig 10G**).

**Fig 10:** Histopathological examination of liver tissue sections in each group. (**A**) Control healthy showing normal hepatocytic cords with normal hepatic cells (Black arrows) and with clear central vein (Red arrows) (H&E, X400); (**B**) HCC-induced showing complete hepatocellular carcinoma, the hepatic tissue is necrotic and occupied by mononuclear cells infiltration (Black arrows) and pyknotic nucleus (orange arrows) and congested dilated portal tracts along with hemorrhage (Red arrows), and dilated sinusoids in between (yellow arrows) (H&E, X400); (**C**) HCC-Bee venom (1 mg/kg) showing focal area of hepatic necrosis occupied by pyknotic nucleus (Green arrows) and congested dilated portal tracts along with hemorrhage (Red arrows), and dilated sinusoids in between (Blue arrows), and all hepatocytes suffer from vacuolar and hydropic degeneration (Black arrows) (H&E, X400); (**D**) HCC-Bee venom (2 mg/kg) showing hepatic tissue is necrotic and occupied by mononuclear cells infiltration (Black arrows) and pyknotic nucleus (orange arrows) and congested dilated portal tracts along with hemorrhage (Red arrows), and dilated sinusoids in between (yellow arrows) (H&E, X400); (**E**) HCC-Targeted bee venom-CSNPs (0.5 mg/kg) showing clear central vein (Red arrows) and almost normal hepatocyte with some hepatocytes suffer from vacuolar and hydropic degeneration (Black arrows) (H&E, X400); (**F**) HCC-Targeted bee venom-CSNPs (1 mg/kg) showing central vein with some hemorrhage (Red arrows) and almost normal hepatocyte with some hepatocytes suffer from vacuolar and hydropic degeneration (Black arrows) (H&E, X400); (**G**) HCC-Non-targeted CSNPs (2 mg/kg) showing focal area of hepatic necrosis occupied by pyknotic nucleus (Black arrows) and larger degenerated area occupied by centrilobular congestion and congested dilated portal tracts along with hemorrhage (Red arrows), and dilated sinusoids in between (yellow arrows).

The article "Bee venom-loaded EGFR-targeting peptide-coupled chitosan nanoparticles for effective therapy of hepatocellular carcinoma by inhibiting EGFR-mediated MEK/ERK pathway" was retracted in 2023. Reasons: concerns about the data; concerns about the images.

## Discussion

The current study is a preliminary attempt to use a freely available existing polymer, chitosan, to improve the pharmacotherapeutic efficacy of a naturally occurring anticancer agent, bee venom, and its smart delivery method against a hepatocellular carcinoma cell. The major goal here is to create a nano-formulation platform capable of reaching the desired site of action by the use of a specific GE11 peptide against overexpressed EGFR receptors. The goal of this somewhat invasive medication delivery technique is to deliver, localize, and extend the release of the bee venom-loaded chitosan nanoparticles (CSNPs) [32]. The EGFR receptor is one such surface receptor that has long been recognized to overexpress the surface of the majority of cancer tumors and has been extensively examined and defined in liver cancer [33]. Targeting EGFR is, therefore, a reasonable method, and to that goal, we derivatized the CSNPs backbone with heterobifunctional PEG, which maintained the particle’s stability profile while also increasing its surface positive charge, allowing it to bind the particular GE11 peptide [34]. The enhanced tumor selectivity was obtained by functionalizing the GE11 peptide of the liver cancer-specific EGFR.

The article "Bee venom-loaded EGFR-targeting peptide-coupled chitosan nanoparticles for effective therapy of hepatocellular carcinoma by inhibiting EGFR-mediated MEK/ERK pathway" was retracted in 2023. Reasons: concerns about the data; concerns about the images.

The data obtained from Zetasizer revealed that targeted bee venom-CSNPs had larger sizes; this might be due to the increased molecular weight of bee venom and composited structure after GE11 addition [35]. In addition, the burst release is thought to be dependent on bee venom dissociation from the formulation, as previously described from loaded protein molecules on CSNPs [36, 37]. Furthermore, the indisputable early quick release and dispersion of protein molecules from the surface of nanoparticles was stated [38]. As a result, the prolonged release of bee venom was linked to the slow breakdown of encapsulated protein molecules as well as the disintegration of nanoparticles themselves [39]. The degradation rate of protein was supposed to exceed its releasing rate, after a prolonged releasing period [40].

We discovered from the obtained results that the method of using GE11-CSNPs as a carrier could be a highly effective way to improve the efficacy and selectivity of bee venom toward HepG2 than SMMC-7721 cells. Previously, it has been observed that the reduced uptake of bee venom is due to resistance caused by the P-glycoprotein pump, which is extensively expressed in cancer and works as an energetic drug efflux pump, resulting in a decrease in cytotoxic protein accumulation [41, 42]. The P-glycoprotein pump is bypassed by the nanoparticle conjugation technique because its uptake is mediated by a particular GE11 peptide that targets the EGFR receptor on liver cancer cells. Thus, surface-modified targeted bee venom-CSNPs were preferentially delivered inside the cells, eliciting a better therapeutic effect than native bee venom, where chitosan and PEG were able to bypass the endosomes, providing a high potential for nuclear delivery.

As we know, surface modification of nano-formulations with specific peptides to enable specific targeting could be a viable technique for increasing therapeutic selectivity against cancer cells, leading to higher drug content at the tumor site, resulting in improved anticancer potentials, and reduced off-target effects [43]. Further, the colony formation experiment demonstrated that, in addition to its anti-proliferative and cytotoxic effects, targeted bee venom-CSNPs efficiently ablated the ability of HepG2 cells to form colonies more than SMMC-7721 cells [44, 45]. Because this experiment analyzes tumor cells’ ability to proliferate and form foci in the absence of growth contact inhibition, it adds to the evidence demonstrating the anticancer potential of targeted bee venom nano-formulation [46].

The article "Bee venom-loaded EGFR-targeting peptide-coupled chitosan nanoparticles for effective therapy of hepatocellular carcinoma by inhibiting EGFR-mediated MEK/ERK pathway" was retracted in 2023. Reasons: concerns about the data; concerns about the images.

There is substantial evidence that most anticancer medicines either directly cause DNA damage or indirectly cause secondary stress-responsive pathways like ROS generation to activate the mitochondrial apoptotic pathway, resulting in apoptosis [47] and inhibiting HepG2 proliferation [48, 49]. For that purpose, we measured the levels of intracellular ROS after treatments with targeted bee venom-CSNPs. When there is an excess of ROS created within the cells, oxidative stress can occur, which can trigger the early stages of apoptosis [48]. Indeed, the anticancer efficacy of bee venom was found to be predominantly dependent on close contact between its active ingredients and cancer cells, which is required to induce cell apoptosis/necrosis [50]. Melittin has been confirmed as a potent bioactive agent for cancer therapy [51]. The main proposed functions of melittin include cell membrane perturbation (resulting in hemolytic and antimicrobial consequences) and the induction of structural alterations including pore formation, vesiculation, and fusion in these membranes [52]. In addition, it promotes tumor cell cycle arrest, limiting proliferation, and death in several tumor cells [53].

As previously reported, bee venom reduced cancer cell proliferation in prostate carcinoma cells besides activation of caspase pathway in xenograft model by inhibition of putative activation of NF-κB activity [54]. In addition, it promotes powerful and highly selective cell death in TNBC and HER2-enriched breast cancer and also MDA-MB-231 [55, 56]. On HepG2, bee venom and melittin exhibit a synergistic anticancer impact with Sorafenib, suggesting a potential HCC therapeutic method [57].‏ Also, melittin inhibits tumor cell metastasis by lowering cell motility and migration via the Rac1-dependent pathway, also due to its strong anti-tumor effectiveness and improved biological safety, melittin nano-liposomes would be a good choice for HCC therapy [58]. In addition to this, bee venom promotes apoptosis in pancreatic cancer cells [59].

In addition, anti-apoptotic Bcl-2 and pro-apoptotic Bax genes are two of the key regulators of the mitochondrial apoptosis process [60]. Indeed, most types of apoptotic cell death are inhibited by Bcl2, suggesting a common lethal mechanism. Bcl2 is found in mitochondria and nuclear membranes, an intracellular source of oxygen-free radical formation. Also, Bcl-2 protected cells from oxidative damage caused by H_2_O_2_ and the overexpression of Bcl-2 completely suppressed lipid peroxidation. Further, Bcl-2 family proteins are distinguished by their capacity to create a complicated combination of heterodimers with Bax and homodimers with themselves [61]. The current findings are comparable to those of Siu-Wan et al [62], who revealed that bee venom can trigger apoptosis in human cervical carcinoma by boosting Bax gene levels while lowering Bcl-2 levels. In addition, Jo et al [63] investigated the inhibition of human ovarian cancer cell growth by bee venom and discovered that expression of pro-apoptotic proteins such as caspase-3, 8, and Bax was increased while Bcl-2 expression was inhibited. Furthermore, it was found that bee venom decreased the expression of Bcl-2 while increasing the expression of Bax, caspase-3, caspase-8, and caspase-9 in colon cancer, which are regulated by NF-κB [64]. Finally, our findings show that targeted bee venom-CSNPs can increase the apoptotic potential of liver cancer cell lines more than native bee venom. As well, caspases, a cysteine protease family, are key initiators and executors of the apoptotic process [65]. At present, the apoptotic pathway was mainly defined as extrinsic and intrinsic. Caspase-9 has been found as an indication of mitochondria-dependent apoptosis pathways, and caspase-3 has been identified as an apoptosis downstream effector caspase [66]. Our results imply that targeted bee venom-CSNPs might trigger HepG2 cell death in a mitochondria-dependent manner.

The article "Bee venom-loaded EGFR-targeting peptide-coupled chitosan nanoparticles for effective therapy of hepatocellular carcinoma by inhibiting EGFR-mediated MEK/ERK pathway" was retracted in 2023. Reasons: concerns about the data; concerns about the images.

Interestingly, the overexpression and phosphorylation of EGFR, which are prevalent mechanisms in epithelial malignancies, are linked to poor prognosis, metastasis, and resistance to chemotherapy, making it a suitable target for cancer treatment [67]. Indeed, the activation of the EGFR-downstream signaling pathway is highly associated with cell protection from apoptosis [68]. We discovered that targeted bee venom-CSNPs blocked the EGFR-mediated proliferation pathway by upregulating pro-apoptotic Bax and downregulating Bcl-2. Furthermore, the conventional EGFR downstream MEK/ERK pathway is a critical signal transduction pathway of cell proliferation [69]. Our findings suggested that targeted bee venom-CSNPs promoted cell death in HepG2 cells via blocking the EGFR-mediated MEK/ERK pathway.

Previous research has shown that inducing cell cycle arrest and death are ideal strategies for cancer treatment [70, 71]. These activities are regulated by a variety of intracellular protein kinases, including MAPKs, which play important roles in cell growth, survival, and apoptosis [72–74]. The p38-MAPK cascade is known to be involved in the apoptotic pathway of human cell lines. Too, human cells exhibit decreased p38-MAPK activity when compared to non-tumorous liver tissue, implying that reduction of p38-MAPK activity causes resistance to apoptosis in human cells. Activation of p38-MAPK has been linked to an apoptotic response generated by numerous anticancer drugs [75]. To the best of our knowledge, no research has been conducted on the relationship between bee venom, the MAPK signaling system, and HepG2 proliferation. Thus, in bee venom-treated HepG2 cells, p38-MAPK activation was studied. Targeted bee venom-CSNPs induce apoptosis in HepG2 cells via activating p38-MAPK and inhibiting MEK/ERK. These findings show that p38-MAPK is involved in bee venom-induced apoptosis in HepG2 cells. As well, various research has indicated that natural compounds like bee venom have a multipotential influence on signaling pathways, including the MAPK pathway. These effects were accompanied by increased phosphorylation of p38-MAPK [76]. As a result, natural chemical bee venom may have numerous regulatory potentials on the MAPK pathway to carry out its anti-tumor impact.

The article "Bee venom-loaded EGFR-targeting peptide-coupled chitosan nanoparticles for effective therapy of hepatocellular carcinoma by inhibiting EGFR-mediated MEK/ERK pathway" was retracted in 2023. Reasons: concerns about the data; concerns about the images.

To evaluate the anti-tumor activity and systemic toxicity of targeted bee venom-CSNPs, we used varying doses of targeted bee venom-CSNPs and native bee venom in the HCC-induced mice model, which is a significant index for its future medical potential. The development of HCC resulted in a significant increase in alpha-fetoprotein levels in our study. Alpha-fetoprotein is one of the most widely utilized diagnostic tumor markers for HCC, and it’s used for tumor diagnosis, monitoring, and even detecting recurrence [77]. The current results indicate that this novel formula has specific anticancer activity against hepatocellular carcinoma in mice.

Furthermore, the damage caused by HCC induction causes the cell membrane of liver tissue to be destroyed, allowing phosphatase and transaminases to escape from the liver into the bloodstream [78]. The obtained results illustrate the novel formula’s ability to retain cell membrane integrity while also repairing the liver injury, preventing carcinogenesis from progressing. The induction of HCC affected the serum levels of albumin and total protein in the current investigation, indicating a severe reduction in hepatic protein production [79]. The injection of DEN causes the dissociation of polyribosomes, which disrupts protein production in the liver [80].

Interestingly, caspase-3, Caspase-9, and Bax expressions were significantly reduced in the DEN-induced mice, but targeted bee venom-CSNPs showed an outstanding increase in these pro-apoptotic genes than native bee venom [81]. Furthermore, overexpression of MMP-9 and MMP-2 was identified in the HCC-induced groups, which is consistent with Chang et al’s findings that DEN therapy elevated MMP-9 and MMP-2 levels as compared to the control group [82]. In DEN-induced mice treated with targeted bee venom-CSNPs, the MMP-9 and MMP-2 genes were dramatically downregulated than native bee venom [83]. Furthermore, the increased expression of the Bcl-2 gene in the liver of HCC-induced mice is consistent with previous research showing that overexpression slows apoptosis and is linked to lower Caspase-3 and Caspase-9 levels in DEN-induced animals [82, 84].

The article "Bee venom-loaded EGFR-targeting peptide-coupled chitosan nanoparticles for effective therapy of hepatocellular carcinoma by inhibiting EGFR-mediated MEK/ERK pathway" was retracted in 2023. Reasons: concerns about the data; concerns about the images.

Furthermore, the higher effectiveness of targeted bee venom-CSNPs was also confirmed by histopathological alterations of treated mice. The targeted bee venom-CSNPs treated cancerous hepatocytes revealed a noticeable recovery and were able to restore the cellular architecture to normal form than native bee venom and are consistent with other *in vivo* and *in vitro* work. Finally, as a result of the current findings, **Fig 11** schematically represents the prospective mechanisms of action of targeted bee venom-CSNPs.

**Fig 11:** Schematic representation of the different pathways for targeted bee venom-CSNPs inside cells.

## Conclusions

In conclusion, we showed that the synthesis of targeted bee venom-CSNPs can improve anti-hepatocellular carcinoma efficacy by targeting cancer cells. GE11 peptide surface modification dramatically increased cellular uptake of nano-formulation via EGFR-mediated endocytosis in EGFR overexpressed cancer cells, resulting in greater inhibitory effects against cancer cells than native bee venom. By increasing ROS production, activating mitochondrial-dependent pathways, blocking EGFR-mediated tyrosine kinase cascades, enhancing p38-MAPK, and blocking the EGFR-mediated tyrosine kinase cascades, targeted bee venom-CSNPs have been discovered to promote cancer cell death.

This cancer-targeted design of bee venom-CSNPs presents a new technique for treating liver cancer *in vitro* and *in vivo* with greater efficacy and fewer side effects than native bee venom, implying that targeted bee venom-CSNPs should be studied further as a chemotherapeutic agent for human malignancies, particularly EGFR over-expressed tumors. In addition, our findings suggest a novel strategy for increasing the value of bee venom.

## Supporting information

S1 Raw images (PDF)

## References

[1] LlovetJM, Zucman-RossiJ, PikarskyE, SangroB, SchwartzM, ShermanM, et al. Hepatocellular carcinoma. Nat Rev Dis Primers. 2016; 2:16018.‏ doi: 10.1038/nrdp.2016.18 27158749

[2] BerasainC, PerugorriaMJ, LatasaMU, CastilloJ, GoniS, SantamariaM, et al. The epidermal growth factor receptor: a link between inflammation and liver cancer. Exp Biol Med. 2009;234:713–725.‏ doi: 10.3181/0901-MR-12 19429859

The article "Bee venom-loaded EGFR-targeting peptide-coupled chitosan nanoparticles for effective therapy of hepatocellular carcinoma by inhibiting EGFR-mediated MEK/ERK pathway" was retracted in 2023. Reasons: concerns about the data; concerns about the images.

[3] JuraN, ZhangX, EndresNF, SeeligerMA, SchindlerT, KuriyanJ. Catalytic control in the EGF receptor and its connection to general kinase regulatory mechanisms. Mol cell. 2001;42:9–22.‏10.1016/j.molcel.2011.03.004PMC317542921474065

[4] LlovetJM, BruixJ. Molecular targeted therapies in hepatocellular carcinoma. Hepatology. 2008;48:1312–1327.‏ doi: 10.1002/hep.22506 18821591PMC2597642

[5] KaufmanNE, DhingraS, JoisSD, VicenteMDGH. Molecular Targeting of Epidermal Growth Factor Receptor (EGFR) and Vascular Endothelial Growth Factor Receptor (VEGFR). Molecules. 2021;26:1076.‏ doi: 10.3390/molecules26041076 33670650PMC7922143

[6] ItoY, TakedaT, HigashiyamaS, SakonM, WakasaKI, TsujimotoM, et al. Expression of heparin binding epidermal growth factor-like growth factor in hepatocellular carcinoma: an immunohistochemical study. Oncol Rep. 2001;8:903–907.‏ doi: 10.3892/or.8.4.903 11410807

[7] LiCM, HaratipourP, LingemanRG, PerryJJP, GuL, HickeyRJ, et al. Novel Peptide Therapeutic Approaches for Cancer Treatment. Cells. 2021;10:2908.‏ doi: 10.3390/cells10112908 34831131PMC8616177

[8] HuhJE, BaekYH, LeeMH, ChoiDY, ParkDS, LeeJD. Bee venom inhibits tumor angiogenesis and metastasis by inhibiting tyrosine phosphorylation of VEGFR-2 in LLC-tumor-bearing mice. Cancer Lett. 2010;292:98–110.‏ doi: 10.1016/j.canlet.2009.11.013 20188461

[9] KhalilA, ElesawyBH, AliTM, AhmedOM. Bee Venom: From Venom to Drug. Molecules. 2021;26:4941. doi: 10.3390/molecules26164941 34443529PMC8400317

[10] YaacoubC, RifiM, El-ObeidD, MawlawiH, SabatierJM, CoutardB, et al. The Cytotoxic Effect of Apis mellifera Venom with a Synergistic Potential of Its Two Main Components-Melittin and PLA2-On Colon Cancer HCT116 Cell Lines. Molecule. 2021;26:2264 doi: 10.3390/molecules26082264 33919706PMC8070685

[11] OršolićN. Bee venom in cancer therapy. Cancer Metastasis Rev. 2012;31:173–194.‏ doi: 10.1007/s10555-011-9339-3 22109081

[12] ParkJH, KimKH, KimSJ, LeeWR, LeeKG, ParkKK. Bee venom protects hepatocytes from tumor necrosis factor-α and actinomycin D. Arch Pharm Res. 2010;33:215–223.‏ doi: 10.1007/s12272-010-0205-6 20195821

[13] TariqR, LiaqatA, KhalidUA. An Insight into the Role of Bee Venom and Melittin Against Tumor Cells: A Review of Breast Cancer therapy. Arch Breast Cancer. 2021;267–276.‏

[14] PutzT, RamonerR, GanderH, RahmA, BartschG, ThurnherM. Antitumor action and immune activation through cooperation of bee venom secretory phospholipase A2 and phosphatidylinositol-(3, 4)-bisphosphate. Cancer Immunol Immunother. 2006;55:1374–1383.‏ doi: 10.1007/s00262-006-0143-9 16485125PMC11030777

[15] GuoH, LiF, QiuH, ZhengQ, YangC, TangC, et al. Chitosan-based nanogel enhances chemotherapeutic efficacy of 10-hydroxycamptothecin against human breast cancer cells. Int J Polym Sci. 2019;2019.‏

The article "Bee venom-loaded EGFR-targeting peptide-coupled chitosan nanoparticles for effective therapy of hepatocellular carcinoma by inhibiting EGFR-mediated MEK/ERK pathway" was retracted in 2023. Reasons: concerns about the data; concerns about the images.

[16] RizeqBR, YounesNN, RasoolK, NasrallahGK. Synthesis, bioapplications, and toxicity evaluation of chitosan-based nanoparticles. Int J Mol Sci. 2019;20:5776.‏10.3390/ijms20225776PMC688809831744157

[17] KirpotinDB, DrummondDC, ShaoY, ShalabyMR, HongK, NielsenUB. et al. Antibody targeting of long-circulating lipidic nanoparticles does not increase tumor localization but does increase internalization in animal models. Cancer Res. 2006;66:6732–6740.‏ doi: 10.1158/0008-5472.CAN-05-4199 16818648

[18] NarmaniA, JafariSM. Chitosan-based nanodelivery systems for cancer therapy: Recent advances. Carbohydr Polym. 2021;272:118464 doi: 10.1016/j.carbpol.2021.118464 34420724

[19] AlconcelSN, BaasAS, MaynardHD. FDA-approved poly (ethylene glycol)–protein conjugate drugs. Polym Chem. 2011;2:1442–1448.‏

[20] BentonAW, MorseRA, StewartJB. Venom collection from honeybees. Science. 1963;142:228–230. doi: 10.1126/science.142.3589.228 17834840

[21] BrandeburgoMAM. A Safe Device For Extracting venom from honeybees. Bee world 1992;73:128–130.

[22] Fakhim-ZadenK. Improved device for venom extraction. Bee world. 1998;79:52–56.‏

[23] BradfordM. A rapid and sensitive method for the quantitation of microgram quantities of protein utilizing the principle of protein-dye binding. Anal Biochem. 1976;72:248–54 doi: 10.1006/abio.1976.9999 942051

[24] GerlierD, ThomassetN. Use of MTT colorimetric assay to measure cell activation. J Immunol Methods. 1986;94:57–63. doi: 10.1016/0022-1759(86)90215-2 3782817

[25] JustusCR, LefflerN, Ruiz-EchevarriaM, YangLV. *In vitro* cell migration and invasion assays. J Vis Exp. 2014;88:51046 doi: 10.3791/51046 24962652PMC4186330

[26] FrankenN, RodermondH, StapJ, HavemanJ, BreeC. Clonogenic assay of cells *in vitro*. Nat Protoc. 2006;1:2315–2319. doi: 10.1038/nprot.2006.339 17406473

[27] GuzmanC, BaggaM, KaurA, WestermarckJ, AbankwaD. Colony Area: an ImageJ plugin to automatically quantify colony formation in clonogenic assays. PloS one. 2014;9:e92444 doi: 10.1371/journal.pone.0092444 24647355PMC3960247

[28] QiSN, YoshidaA, WangZR, UedaT. GP7 can induce apoptotic DNA fragmentation of human leukemia cells through caspase-3-dependent and -independent pathways. Int J Mol Med. 2004;13:163–167 14654989

[29] LivakK, SchmittgenT. Analysis of relative gene expression data using real-time quantitative PCR and the 2(-Delta Delta C(T)) method. Methods. 2001;25:402–8 doi: 10.1006/meth.2001.1262 11846609

[30] BurnetteW. Western blotting: electrophoretic transfer of proteins from sodium dodecyl sulfate-polyacrylamide gels to unmodified nitrocellulose and radiographic detection with antibody and radioiodinated protein A. Anal Biochem. 1981;112:195–203. doi: 10.1016/0003-2697(81)90281-5 6266278

The article "Bee venom-loaded EGFR-targeting peptide-coupled chitosan nanoparticles for effective therapy of hepatocellular carcinoma by inhibiting EGFR-mediated MEK/ERK pathway" was retracted in 2023. Reasons: concerns about the data; concerns about the images.

[31] BancroftJD, StevensA. Theory and Practice of Histological Techniques, 4th ed. Churchill Livingston, New York, Edinburgh, London;1996.

[32] HaiderN, FatimaS, TahaM, RizwanullahM, FirdousJ, AhmadR, et al. Nanomedicines in di-agnosis and treatment of cancer: an update. Curr Pharm Design. 2020;26:1216–1231.10.2174/138161282666620031817071632188379

[33] ZandiR, LarsenAB, AndersenP, StockhausenMT, PoulsenHS. Mechanisms for oncogenic activation of the epi-dermal growth factor receptor. Cell Signal. 2007;19:2013–2023.‏ doi: 10.1016/j.cellsig.2007.06.023 17681753

[34] ShiL, ZhangJ, ZhaoM, TangS, ChengX, ZhangW, et al. Effects of polyethylene glycol on the surface of nanoparticles for targeted drug delivery. Nanoscale. 2021;13:10748–10764. doi: 10.1039/d1nr02065j 34132312

[35] SoaresKSR, FonsecaJLC, BitencourtMAO, SantosKS, Silva-JúniorAA, Fernandes-PedrosaMF. Serum pro-duction against *Tityus serrulatus* scorpion venom using cross-linked chitosan nanoparticles as immunoadjuvant. Toxicon. 2012;60:1349–1354.‏ doi: 10.1016/j.toxicon.2012.09.010 23006936

[36] JarudilokkulS, TongthammachatA, BoonamnuayvittayaV. Preparation of chitosan nanoparticles for encapsulation and release of protein. Korean J Chem Eng. 2011;28:1247–1251.‏

[37] GanQ, WangT, CochraneC, McCarronP. Modulation of surface charge, particle size and morphological properties of chitosan–TPP nanoparticles intended for gene delivery. Colloids Surf B Biointerfaces. 2005;44:65–73.‏ doi: 10.1016/j.colsurfb.2005.06.001 16024239

[38] ZhouS, DengX, LiX. Investigation on a novel core-coated microspheres protein delivery system. J Control Release. 2001;75:27–36.‏ doi: 10.1016/s0168-3659(01)00379-0 11451494

[39] ZhouS, DengX, YuanM, LiX. Investigation on preparation and protein release of biodegradable polymer micro-spheres as drug‐delivery system. J Appl Polym Sci. 2002;84:778–784.‏

[40] AmidiM, RomeijnSG, BorchardG, JungingerHE, HenninkWE, JiskootW. Preparation and characterization of protein-loaded N-trimethyl chitosan nanoparticles as nasal delivery system. J Control Release. 2006;111:107–116.‏ doi: 10.1016/j.jconrel.2005.11.014 16380189

[41] HuiRC, FrancisRE, GuestSK, CostaJR, GomesAS, MyattSS, et al. Doxorubicin activates FOXO3a to induce the expression of multidrug resistance gene ABCB1 (MDR1) in K562 leukemic cells. Mol Cancer Ther. 2008;7:670–678. doi: 10.1158/1535-7163.MCT-07-0397 18347152

[42] SahooSK, LabhasetwarV. Enhanced anti-proliferative activity of transferring conjugated paclitaxel loaded nanoparticle is mediated via sustained intracellular drug retention. Mol Pharm. 2005;2:373–383. doi: 10.1021/mp050032z 16196490

The article "Bee venom-loaded EGFR-targeting peptide-coupled chitosan nanoparticles for effective therapy of hepatocellular carcinoma by inhibiting EGFR-mediated MEK/ERK pathway" was retracted in 2023. Reasons: concerns about the data; concerns about the images.

[43] FuX, ShiY, QiT, QiuS, HuangY, ZhaoX, et al. Precise design strategies of nanomedicine for improving cancer therapeutic efficacy using subcellular targeting. Signal Transduct Target Ther. 2020;5:262. doi: 10.1038/s41392-020-00342-0 33154350PMC7644763

[44] LimHN, BaekSB, JungHJ. Bee venom and its peptide component melittin suppress growth and migration of melanoma cells via inhibition of PI3K/AKT/mTOR and MAPK pathways. Molecules. 2019;24:929. doi: 10.3390/molecules24050929 30866426PMC6429308

[45] ChoiKE, HwangCJ, GuSM, ParkMH, KimJH, ParkJH, et al. Cancer cell growth inhibitory effect of bee venom via increase of death receptor 3 expression and inactivation of NF-kappa B in NSCLC cells. Toxins. 2014;6:2210–2228. doi: 10.3390/toxins6082210 25068924PMC4147578

[46] ZhangGS, TuCQ, ZhangGY, ZhouGB, ZhengWL. Indomethacin induces apoptosis and inhibits proliferation in chronic myeloid leukemia cells. Leuk Res. 2000;24:385–392 doi: 10.1016/s0145-2126(99)00198-8 10785260

[47] KhanN, AfaqF, MukhtarH. Apoptosis by dietary factors: The suicide solution for delaying cancer growth. Carcinogenesis. 2007;28:233–9 doi: 10.1093/carcin/bgl243 17151090

[48] OttM, GogvadzeV, OrreniusS, ZhivotovskyB. Mitochondria, oxidative stress and cell death. Apoptosis. 2007;12:913–22 doi: 10.1007/s10495-007-0756-2 17453160

[49] MadejaZ, SrokaJ, NyströmC, Björkhem-BergmanL, NordmanT, DamdimopoulosA, et al. The role of thioredoxin reductase activity in selenium-induced cytotoxicity. Bio-chem Pharmacol. 2005;69:1765–72. doi: 10.1016/j.bcp.2005.02.023 15935149

[50] OršolićN, ŠverL, VerstovšekS, TerzićS, BašićI. Inhibition of mammary carcinoma cell proliferation *in vitro* and tumor growth *in vivo* by bee venom. Toxicon. 2003;41:861–870 doi: 10.1016/s0041-0101(03)00045-x 12782086

[51] DempseyCE. The actions of melittin on membranes. Biochim Biophys Acta Biomembr. 1990;1031:143–161.‏ doi: 10.1016/0304-4157(90)90006-x 2187536

[52] LeuschnerC, HanselW. Membrane disrupting lytic peptides for cancer treatments. Curr Pharm Des. 2004;10:2299–2310.‏ doi: 10.2174/1381612043383971 15279610

[53] OršolićNADA, ŠverL, BendeljaK, BašićI. Antitumor activity of bee venom. Period Biol. 2001;103:49

[54] ParkMH, ChoiMS, KwakDH, OhKW, Yoon doY, HanSB, et al. Anti-cancer effect of bee venom in prostate cancer cells through activation of caspase pathway via inactivation of NF-kappaB. Prostate. 2011;71:801–812. doi: 10.1002/pros.21296 21456063

[55] DuffyC, SorollaA, WangE, GoldenE, WoodwardE, DavernK, et al. Honeybee venom and melittin suppress growth factor receptor activation in HER2-enriched and triple-negative breast cancer. NPJ Precis Oncol. 2020;24:1–16 doi: 10.1038/s41698-020-00129-0 32923684PMC7463160

The article "Bee venom-loaded EGFR-targeting peptide-coupled chitosan nanoparticles for effective therapy of hepatocellular carcinoma by inhibiting EGFR-mediated MEK/ERK pathway" was retracted in 2023. Reasons: concerns about the data; concerns about the images.

[56] JungGB, HuhJE, LeeHJ, KimD, LeeGJ, ParkHK, et al. Anti-cancer effect of bee venom on human MDA-MB-231 breast cancer cells using Raman spectroscopy. Biomed Opt Express. 2018;9:5703–5718 doi: 10.1364/BOE.9.005703 30460157PMC6238932

[57] MansourGH, El-MagdMA, MahfouzDH, AbdelhamidIA, MohamedMF, IbrahimNS, et al. Bee venom and its active component Melittin synergistically potentiate the anticancer effect of Sorafenib against HepG2 cells. Bioorg Chem. 2021;116:105329 doi: 10.1016/j.bioorg.2021.105329 34544028

[58] MaoJ, LiuS, AiM, WangZ, WangD, LiX, et al. A novel melittin nano-liposome exerted excellent anti-hepatocellular carcinoma efficacy with better biological safety. J Hematol Oncol. 2017; 10:71.‏ doi: 10.1186/s13045-017-0442-y 28320480PMC5359812

[59] ZhaoJ, HuW, ZhangZ, ZhouZ, DuanJ, DongZ, et al. Bee venom protects against pancreatic cancer via inducing cell cycle arrest and apoptosis with suppression of cell migration. J Gastrointest Oncol. 2022;13: 847–858.‏ doi: 10.21037/jgo-22-222 35557571PMC9086033

[60] TongQS, ZhengLD, WangL, LiuJ, QianW. BAK overexpression mediates p53-independent apoptosis inducing effects on human gastric cancer cells. BMC Cancer. 2004;4:33. doi: 10.1186/1471-2407-4-33 15248898PMC481072

[61] ReedJC. Double identity for proteins of the Bcl-2 family. Nature. 1997;387:773–776 doi: 10.1038/42867 9194558

[62] IpSW, WeiHC, LinJP, KuoHM, LiuKC, HsuSC, et al. Bee venom induced cell cycle arrest and apoptosis in human cervical epidermoid carcinoma Ca Ski cells. Anticancer Res. 2008;28:833–42. 18507026

[63] JoM, ParkMH, KolliparaPS, AnBJ, SongHS, HanSB, et al. Anti-cancer effect of bee venom toxin and melittin in ovarian cancer cells through induction of death receptors and inhibition of JAK2/STAT3 pathway. Toxicol Appl Pharmacol. 2012;258:72–81 doi: 10.1016/j.taap.2011.10.009 22027265

[64] ZhengJ, LeeHL, HamYW, SongHS, SongJ, HongJT. Anti-cancer effect of bee venom on colon cancer cell growth by activation of death receptors and inhibition of nuclear factor kappa B. Oncotarget. 2015;6:44437–44451 doi: 10.18632/oncotarget.6295 26561202PMC4792567

[65] ShaliniS, DorstynL, DawarS, KumarS. Old, new and emerging functions of caspases. Cell Death Differ. 2015;22:526–539‏ doi: 10.1038/cdd.2014.216 25526085PMC4356345

[66] AdamsJM. Ways of dying: multiple pathways to apoptosis. Genes Dev. 2003;17:2481–95 doi: 10.1101/gad.1126903 14561771

[67] NicholsonRI, GeeJM, HarperME. EGFR and cancer prognosis. Eur J Cancer. 2001;37:S9–S15 doi: 10.1016/s0959-8049(01)00231-3 11597399

[68] NicholsonKM.; AndersonN.G. The protein kinase B/Akt signalling pathway in human malignancy. Cell Signal. 2002;14:381–95 doi: 10.1016/s0898-6568(01)00271-6 11882383

The article "Bee venom-loaded EGFR-targeting peptide-coupled chitosan nanoparticles for effective therapy of hepatocellular carcinoma by inhibiting EGFR-mediated MEK/ERK pathway" was retracted in 2023. Reasons: concerns about the data; concerns about the images.

[69] RooversK, AssoianRK. Integrating the MAP kinase signal into the G1 phase cell cycle machinery. Bioessays. 2000;22:818–26 doi: 10.1002/1521-1878(200009)22:9&lt;818::AID-BIES7&gt;3.0.CO;2-6 10944584

[70] SchwartzGK, ShahMA. Targeting the cell cycle: a new approach to cancer therapy. J Clin Oncol. 2005;23:9408–9421 doi: 10.1200/JCO.2005.01.5594 16361640

[71] ChoMH, KimS, LeeJH, ShinTH, YooD, CheonJ. Magnetic tandem apoptosis for overcoming multidrug-resistant cancer. ‏Nano Lett. 2016;16:7455–7460 doi: 10.1021/acs.nanolett.6b03122 27960458

[72] GaoS, SunD, WangG, ZhangJ, JiangY, LiG, et al. Growth inhibitory effect of paratocarpin E, a prenylated chalcone isolated from *Euphorbia humifusa* Wild., by induction of autophagy and apoptosis in human breast cancer cells. Bioorg Chem. 2016;69:121–128. doi: 10.1016/j.bioorg.2016.10.005 27814565

[73] KimKN, HamYM, MoonJY, KimMJ, JungYH, JeonYJ, et al. Acanthoic acid induces cell apoptosis through activation of the p38 MAPK pathway in HL-60 human promyelocytic leukaemia. Food Chem. 2012;135:2112–7. doi: 10.1016/j.foodchem.2012.05.067 22953963

[74] ChaoJI, YangJL. Opposite roles of ERK and p38 mitogen-activated protein kinases in cadmium-induced genotoxicity and mitotic arrest. Chem Res Toxicol. 2001;14:1193–1202 doi: 10.1021/tx010041o 11559033

[75] CuiY, LuP, SongG, LiuQ, ZhuD, LiuX. Involvement of PI3K/Akt, ERK and p38 signaling pathways in emodin-mediated extrinsic and intrinsic human hepatoblastoma cell apoptosis. Food Chem Toxicol. 2016;92:26–37. doi: 10.1016/j.fct.2016.03.013 27032576

[76] HuhJE, KangJW, NamD, BaekYH, ChoiDY, ParkDS, et al. Melittin suppresses VEGF-A-induced tumor growth by blocking VEGFR-2 and the COX-2-mediated MAPK signaling pathway. J Nat Prod. 2012;75:1922–9. doi: 10.1021/np300446c 23110475

[77] JaganS, RamakrishnanG, AnandakumarP, KamarajS, DevakiT. Antiproliferative potential of gallic acid against diethylnitrosamine-induced rat hepatocellular carcinoma. Mol Cell Biochem. 2008;319:51–59 doi: 10.1007/s11010-008-9876-4 18629614

[78] GianniniEG, TestaR, SavarinoV. Liver enzyme alteration: a guide for clinicians. Can Med Assoc J. 2005;172:367–379 doi: 10.1503/cmaj.1040752 15684121PMC545762

[79] HeidelbergerC. Chemical carcinogenesis. Annu Rev Biochem. 1975;44:79–121. doi: 10.1146/annurev.bi.44.070175.000455 1094923

[80] XiaoB, CuiLM, MaDJ, LiuSP, ZhangXW. Endoplasmic reticulum stress in diethylnitrosamine-induced rat liver cancer. Oncol Lett. 2014;7:23–27. doi: 10.3892/ol.2013.1651 24348814PMC3861556

[81] VedarethinamV, DhanarajK, IlavenilS, ArasuMV, ChoiKC, Al-DhabiNA, et al. Antitumor Effect of the Mannich Base(1,3-bis-((3-Hydroxynaphthalen-2-yl)phenylmethyl)urea) on Hepatocellular Carcinoma. Molecules. 2014;21:63210.3390/molecules21050632PMC627373427187346

The article "Bee venom-loaded EGFR-targeting peptide-coupled chitosan nanoparticles for effective therapy of hepatocellular carcinoma by inhibiting EGFR-mediated MEK/ERK pathway" was retracted in 2023. Reasons: concerns about the data; concerns about the images.

[82] ChangW, HeW, LiPP, SongSS, YuanPF, LuJT, et al. Protective effects of Celastrol on diethylnitrosamine-induced hepatocellular carcinoma in rats and its mechanisms. Eur J Pharmacol. 2016;784:173–80. doi: 10.1016/j.ejphar.2016.04.045 27181068

[83] MałekA, KocotJ, MitrowskaK, PosyniakA, KurzepaJ. Bee venom effect on glioblastoma cells viability and gelatinase secretion. Front Neurosci. 2022;16:792970. doi: 10.3389/fnins.2022.792970 35221898PMC8873382

[84] SabokrouhA, GoodarziMT, Vaisi-RayganiA, KhatamiS, Taghizadeh-JahedM. Effects of treatment with platinum azidothymidine and azidothymidine on telomerase activity and Bcl-2 concentration in hepatocellular carcinoma- induced rats. Avicenna J Med Biotechnol. 2014;6:200–9. 25414782PMC4224659

